The article "Integrative Functional Genomic Analysis in Multiplex Autism Families from Kazakhstan" was published in 2022. Journal: Dis Markers.

# Integrative Functional Genomic Analysis in Multiplex Autism Families from Kazakhstan

**DOI:** 10.1155/2022/1509994

**Published:** 2022-09-26

**Authors:** Anastassiya Perfilyeva, Kira Bespalova, Yuliya Perfilyeva, Liliya Skvortsova, Lyazzat Musralina, Gulnur Zhunussova, Elmira Khussainova, Ulzhan Iskakova, Bakhytzhan Bekmanov, Leyla Djansugurova

**Affiliations:** ^1^Institute of Genetics and Physiology, 93 Al-Farabi Ave., Almaty 050060, Kazakhstan; ^2^Al-Farabi Kazakh National University, 71 Al-Farabi Ave., Almaty 050040, Kazakhstan; ^3^M.A. Aitkhozhin's Institute of Molecular Biology and Biochemistry, 86 Dosmukhamedov St., Almaty 050012, Kazakhstan; ^4^Branch of the National Center for Biotechnology, 14 Zhahanger St., Almaty 050054, Kazakhstan; ^5^Kazakh National Medical University, 94 Tole Bi St., Almaty 050000, Kazakhstan

## Abstract

The study of extended pedigrees containing autism spectrum disorder- (ASD-) related broader autism phenotypes (BAP) offers a promising approach to the search for ASD candidate variants. Here, a total of 650,000 genetic markers were tested in four Kazakhstani multiplex families with ASD and BAP to obtain data on *de novo* mutations (DNMs), common, and rare inherited variants that may contribute to the genetic risk for developing autistic traits. The variants were analyzed in the context of gene networks and pathways. Several previously well-described enriched pathways were identified, including ion channel activity, regulation of synaptic function, and membrane depolarization. Perhaps these pathways are crucial not only for the development of ASD but also for ВАР. The results also point to several additional biological pathways (circadian entrainment, NCAM and BTN family interactions, and interaction between L1 and Ankyrins) and hub genes (CFTR, NOD2, PPP2R2B, and TTR). The obtained results suggest that further exploration of PPI networks combining ASD and BAP risk genes can be used to identify novel or overlooked ASD molecular mechanisms.

## 1. Introduction

ASD is a spectrum of psychological characteristics that describe a wide range of abnormal behavior and difficulties in social cooperation and communication, as well as severely restricted interests and frequently repetitive behaviors. Relevance of the ASD problem arises from the high incidence of this pathology all over the world, including Kazakhstan. According to official data, in 2021, there were 4,887 children with ASD in Kazakhstan, but experts believe that this indicator is ten times higher. According to the statistics of WHO and CDC, there are at least 30,000 children with ASD in Kazakhstan (https://inbusiness.kz/ru/last/v-kazahstane-30-tysyach-detej-stradayut-autizmom).

The article "Integrative Functional Genomic Analysis in Multiplex Autism Families from Kazakhstan" was published in 2022. Journal: Dis Markers.

The etiology of this pathology is extremely difficult and is probably determined by a combination of genetic susceptibility and environmental factors. Determining the specific contribution of these factors to ASD is difficult due to the lack of population-based, longitudinal evidence necessary to establish conclusive links between exposure, genotypic responses, and phenotypic consequences [1]. Some studies steered the debate toward the greater importance of environmental factors rather than a genetic predisposition to ASD [2, 3]. Other studies showed little support for general environmental influences [4, 5]. Most recent studies suggest that environmental exposures may be a catalyst for deleterious DNMs leading to ASD [1], whereas genetic factors are considered the predominant causes of ASD [6, 7]. A strong contribution of heritable factors in the etiology of ASD is supported by twin studies and studies of first-degree relatives. Indeed, the risk of a child being diagnosed with ASD is increased at least 25-fold in a family where a brother or sister has already been diagnosed with autism [8]. Independent twin studies show concordance rates of 60-92% in monozygotic twins versus 0-10% in dizygotic twins [9, 10]. If only one child in a family has ASD, the other twin may have delayed speech, reading, and spelling difficulties [11]. This study by Folstein et al. of siblings and parents of affected children with mild cognitive and behavioral impairments led to the concept of the BAP [11]. Apparently, ASD families with multiple occurrences and relatives with BAP have a higher genetic loading for ASD [12], making them a good model for studies when environmental factors are excluded or have minimal influence. Such families are not uncommon in ASD, and several studies of such pedigrees have been published [13–16]. The prevalence of BAP in ASD families is also not low. A large-scale study by Sasson et al. estimates that the prevalence rate of BAP among parents of children with ASD ranges from 14 to 23% [17]. A meta-analysis of twin studies found that there is no disruption between ASD and BAP in genetic modeling, suggesting that ASD as a disorder can be conceptualized as the extreme of BAP symptoms/behaviors [18]. If this is the case, the inclusion of individuals with BAP in a study of multiplex families should increase the power of the study to determine the genetic structure of ASD [16, 19].

A complex understanding of the genetic structure of ASD requires unbiased knowledge of the number of risk loci, their penetrance, and allele frequencies [19]. The collected data to date provided conclusive evidence for three categories of genetic structure, including common SNPs (MAF > 1%), inherited rare variants (MAF < 1%), and DNMs that have been identified in the proband and are not found in the genome of the biological parents [20]. Genetic models suggest that at least 50% of the variance in ASD may be due to common inherited variants [21], which act in aggregate while having little effect individually. Despite evidence for a significant role of common variants in ASD risk, rare genetic variations may be associated with higher individual risk [22]. Maintenance of genetic susceptibility to ASD despite reduced transmission of risk variants may be due to DNMs [23, 24]. The relative contribution of spontaneous DNMs to the ASD etiology is estimated between 5 and 15% [23]. In several cases of syndromic ASD, a single DNM appears to be sufficient to cause the onset of ASD symptoms [25], suggesting that this DNM disrupts key loss-of-function intolerant genes. Despite a considerable genetic heterogeneity underlying ASD, there is compelling evidence that a large number of risk genes can be integrated into a much smaller number of protein-protein interaction (PPI) networks [26]. Previous studies have shown that ASD genes functionally converge in synapse development, axon alignment, neuron motility, synaptic transmission, chromatin remodeling, transcription and translation regulation, ion transport, and cell adhesion [27–32]. As far as we know, these studies were mainly focused on investigating genes affected in children with ASD, but not in relatives with subclinical phenotypes of BAP. The foregoing suggests that inclusion of ASD-related genes from first-degree relatives with BAP in the PPI network may help to better understand the development of autistic traits in the family. Will the main pathways of development of autistic traits change from those shown so far in this case? If ASD is simply the extreme end of the distribution of autistic traits that make up BAP, there will not be a large shift in the main trajectory. However, will other less studied convergent signaling mechanisms or protein interactions contributing to ASD pathology be identified? The previously discovered BAP genes [33–37] lead to the assumption that BAP gene loci generally correlate with ASD loci. However, several loci were found to be significant only for BAP [13], suggesting that the absence of the BAP putative risk gene in the PPI networks may be a missing link to understanding the initial biological mechanisms of ASD. Therefore, here, we focused on a set of four extended pedigrees with ASD and BAP. The aim of the study was to identify putative candidate genes and to investigate functional relationships between these genes using PPI network analysis. This is the first genetic study of Kazakhstani families with ASD.

The article "Integrative Functional Genomic Analysis in Multiplex Autism Families from Kazakhstan" was published in 2022. Journal: Dis Markers.

## 2. Materials and Methods

### 2.1. Sampling

Families for this study were selected using a database of 400 Kazakhstani families with ASD children. The database was created within the framework of the previously implemented project 0118РК00503 in 2018-2021. We applied the following inclusion criteria for families: two or more children with ASD AND BAP among first-degree relatives AND Kazakhstani ancestry. Exclusion criteria were a simplex family OR/AND fragile X syndrome. A total of 13 families (3%, 95% CI: 1.7-5.5%) met the inclusion and exclusion criteria. Three families were out of the country at the time of the study, two families were single parents, and four families declined to participate in the study for one reason or another. Thus, four families took part in the study. Samples of saliva were collected from all children with ASD as well as from their parents and neurotypical siblings using a collection kit (Zeesan) provided by TellmeGen.

Collection was conducted after obtaining informed consent from at least one of the parents. The study was approved by the Ethics Committee of the Institute of Human and Animal Physiology, Almaty, Kazakhstan. The children recruited in this study were diagnosed with ASD by psychiatrist. The Child Autism Rating Scale (CARS) was used to assess the severity of ASD [38]. The Broad Autism Phenotype Questionnaire (BAPQ) was used to assess BAP traits [39, 40].

### 2.2. Data Generation

DNA isolation from the collected biomaterial and data generation were performed using the Infinium Global Screening Array (GSA) v3.0 run on the Illumina iScan Platform at TellmeGen CA (Valencia, Spain). A total of 650,000 genetic markers were analyzed using 10,000 probes (99.99% reliability). A triplicate analysis was performed.

### 2.3. Data Analysis

Family trees were generated using the GenoPro2020 software (https://genopro.com/2020/).

TellmeGen CA applied standardized quality control measures to filter out low-quality data (a call rate lower than 0.99) from the SNP list and compiled all obtained results into csv files, which were sent to our laboratory for further analysis.

Genetic variants were aligned to the GRCh37 human reference genome and annotated in accordance with the nomenclature of the HGVS (Human Genome Variation Society) [41]. Gene-based annotation was performed using the RStudio software (http://rstudio.com/products/rstudio/) with gene definitions from the database of dbSNP (http://www.ncbi.nlm.nih.gov/projects/SNP/), ClinVar (https://www.ncbi.nlm.nih.gov/clinvar/), SFARI (Simons Foundation Autism Research Initiative, http://gene.sfari.org/), and GWAS catalog (Genome-Wide Association Studies, https://http://www.ebi.ac.uk/gwas/home). The MAF (minor allele frequency) was estimated using the databases ALFA (allele frequency aggregator, http://nih.gov), 1000G (1000 Genomes, http://www.1000genomes.org/), gnomAD (Genome Aggregation, https://gnomad.broadinstitute.org/), andTOPMed (trans-Omics for Precision Medicine, https://www.nhlbi.nih.gov/science/trans-omics-precision-medicine-topmed-program).

The article "Integrative Functional Genomic Analysis in Multiplex Autism Families from Kazakhstan" was published in 2022. Journal: Dis Markers.

The GSA includes ∼640,000 single nucleotide polymorphisms (SNPs) and ∼10,000 indels (insertion/deletion). SNPs that are missing from a fraction of individuals in the cohort were filtered out. SNPs with a MAF > 1% associated with ASD according to the GWAS catalog (*p* < 0.00001) were included in the list of common variants. SNPs with a MAF ≤ 0.01% associated with ASD according to the ClinVar database and inherited by a child with ASD from a parent with BAP were included in the list of rare inherited variants.

DNMs were identified according to the scenario: both parents carry a homozygous reference allele and the child is heterozygous, i.e., carries one copy each of the alleles REF and ALT. The variants were classified as pathogenic, probably pathogenic, of unclear significance (VUS), benign, or probably benign according to the ACMG (American College of Medical Genetics and Genomics) guidelines [12]. Pathogenic mutations included stop codon variants (frameshift and nonsense mutations), variants with uncorrected splicing, and variants with previously established pathogenic effects according to ClinVar database. *In silico* tools such as SIFT (Sorting Intolerant From Tolerant, http://sift-dna.org) and Polymorphism Phenotyping-2 (PolyPhen-2, http://genetics.bwh.harvard.edu/pph2/) were used to predict deleterious effects of missense variants on protein structure and function. We filtered out variants that were most likely nonpathogenic (benign and likely benign) or with MAF < 1% in order to identify clinically relevant rare DNMs.

### 2.4. Data Visualization and Functional Interpretation

To characterize the relationships between the ASD/BAP candidate genes in each family, we projected them into the PPI network. The InnateDB (Knowledge Resource for Innate Immunity Interactions and Pathways, https://www.innatedb.com/) was used to retrieve predicted interactions for the identified candidate genes [42, 43]. The OmicsNet 2.0 software (https://www.omicsnet.ca) was used to construct the PPI network. This is a novel web-based tool for creation and visualization of complex biological networks. The software supports ten molecular interaction databases for protein-protein, miRNA-target, TF-target, and enzyme-metabolite interactions and provides multiple methods for network customization using a powerful WebGL technology to enable native 3D display of complex biological networks in modern web browsers [44]. The WalkTrap algorithm in OmicsNet 2.0 was applied to further partition of the PPI into modules. The algorithm assumes that a random walker tends to be trapped in dense parts of a network corresponding to modules.

The article "Integrative Functional Genomic Analysis in Multiplex Autism Families from Kazakhstan" was published in 2022. Journal: Dis Markers.

Functional annotation and enrichment analysis of genes were performed according to the GO (Gene Ontology, http://geneontology.org/) [45], KEGG (Kyoto Encyclopedia of Genes and Genomes, https://www.genome.jp/kegg), and REACTOME (http://www.reactome.org) databases using the g:Profiler (https://biit.cs.ut.ee/gprofiler/). This is an open web server for characterizing and manipulating gene lists. It is updated every three months following the quarterly releases of the Ensembl databases [46]. The g:Profiler Bonferroni correction was used, and only pathways with an adjusted *p* value (*p*_adj_) < 0.05 were considered significantly enriched.

## 3. Results

### 3.1. Characteristics of Subjects

The study included four multiplex families (Figure 1). The mean age (± standard deviation) of the ASD children was 9.1 ± 4.2 years. The ratio of male to female children with ASD was 7 : 1. The mean ages of parents and neurotypical siblings were 39.3 ± 3.5 and 14.5 ± 7.8 years, respectively.

Family 1 has two boys with moderate ASD and one neurotypical girl. Family 2 has two sons with severe and moderate ASD and one neurotypical daughter. Family 3 has two sons with moderate autism. In Family 4, the mother has two children from different marriages. The son has severe ASD, and the daughter has moderate autism. The BAPQ data indicated that the fathers from Families 1, 2, and 3 and the mothers from Families 2 and 4 have autistic traits with high scores across the domains of ASD. The fathers from Families 1 and 3 and the mother from Family 2 have high aloofness subscale scores, while the father from Family 2 has pragmatic language deficits. The mother from Family 4 has either BAP or ASD and shows rigid personality and pragmatic language deficits. All family members are Kazakh except the father and his daughter from Family 4. They are Russian.

### 3.2. Identification and Annotation of ASD and BAP Associated Variants/Genes

A total of 650,000 genetic markers were analyzed to generate data on DNMs, common, and rare variants that may contribute to autistic traits. A total of 72 common variants associated with ASD were identified, including three regulatory region variants (4.2%), three prime UTR variants (4.2%), 15 intergenic variants (20.8%), 48 intron variants (66.6%), one missense variant (1.4%), one noncoding transcript exon variant (1.4%), and one VUS variant (1.4%). A total of 29 (40%) of 72 common variants overlapped in four pedigrees (Table 1). Further analysis demonstrated 50 rare inherited variants, including 40 missense (80%), three splice donors (6%), five synonymous (10%), and two stop-gain variants (4%). Two rare variants (4%) occurred in all four pedigrees (Table 2).

The article "Integrative Functional Genomic Analysis in Multiplex Autism Families from Kazakhstan" was published in 2022. Journal: Dis Markers.

DNMs were found only in children with ASD but not in neurotypical siblings. In total, 12 heterozygous DNMs were identified in three families, including nine missense variants, two nonsense mutations, and one splice variant (Table 3). No DNMs were detected in Family 3. We found no identical mutations in ASD siblings.

### 3.3. PPI Network and Functional Enrichment Analysis

We prioritized candidate genes 57, 60, 58, and 73 in Families 1, 2, 3, and 4, respectively. The PPI networks for these genes were constructed for each pedigree. As a result, four networks with the following properties were obtained: 614 nodes, 672 edges, and 35 seeds for Family 1, 746 nodes, 870 edges, and 36 seeds for Family 2, 669 nodes, 743 edges, and 39 seeds for Family 3, and 923 nodes, 1092 edges, and 50 seeds for Family 4. After partitioning into modules, these networks were divided into 14 significant modules for Families 1 and 2, 11 modules for Family 3, and 20 modules for Family 4 (Figure 2). The number of connections of a node or the degree of centrality (DC) showed that ten genes, namely HDAC4, CFTR, MECP2, NOD2, PPP2R2B, TCF4, TRIM33, TSC2, TTN, and TTR, play a nodal role in the generated networks and form the largest modules (Table 4). The highest-ranking node in all networks was HDAC4 (DC = 202), except in Family 4, where CFTR played a greater role (DC = 222). In Families 2 and 3, another high-ranking node was TTN (DC = 104). TCF4, PPP2R2B, and HDAC4 were common hub genes for all four networks.

We then assumed that the set of identified genes for each pedigree work together and can be integrated into a single module. We defined them as disease modules and performed the enrichment analysis. A total of 92 enriched terms for Family 1 (18 GO MF, 44 GO BP, 26 GO CC, and 4 REAC), 19 enriched terms for Family 2 (18 GO MF, 44 GO BP, 26 GO CC, and 4 REAC), 37 enriched terms for Family 3 (9 GO MF, 9 GO BP, and 19 GO CC), and 155 enriched terms for Family 4 (29 GO MF, 72 GO BP, 46 GO CC, 7 REAC, and 1 KEGG) were identified. The results of the top 15 terms in each GO category and all results in REACTOME and KEGG are presented in Table 5.

Families 1, 3, and 4 showed very similar patterns of the GO MF pathways. The enriched molecular function in these families was ion channel activity (GO: 0086056, GO: 0005245, GO: 0086007, GO: 0022836, GO: 0005216, GO: 0005244, GO: 0022832, and GO: 0015267). In Family 2, interleukin-1 receptor activity (IL-1) (GO: 0004908) and binding (GO: 0019966), cation transmembrane transporter (GO: 0008324), and gated channel activity (GO: 0022836) were enriched. In the BP category, candidate genes were mainly enriched in biological processes, such as membrane depolarization (GO: 0086010, GO: 0051899, GO: 0086012, GO: 0098912, and GO: 0086045) and regulation of synaptic functions (anterograde transsynaptic signaling GO: 0098916, chemical synaptic transmission GO: 0007268, transsynaptic signaling GO: 0099537, and synaptic signaling GO: 0099536). In addition, the processes of reactive oxygen biosynthesis (GO: 1903409, GO: 1903426) and ion transport (GO: 0034220, GO: 0006812) were enriched in Family 2. In the CC category, candidate genes were enriched in synapses (GO: 0097060, GO: 0045211, GO: 0098794, GO: 0045202, and GO: 0098978) and ion channel complexes (GO: 0005891, GO: 0034704, GO: 1990454, GO: 0034702, and GO: 0034703). In Family 2, candidate genes were also found in the node of Ranvier (GO: 0033268) and in the initial segment of the axon (GO: 0043194). A significant KEGG pathway associated with circadian control (KEGG: 04713) was found in Family 4. The most significant REACTOME pathways included NCAM1 interactions (REAC: R-HSA-419037) and signaling for neurite out-growth (REAC: R-HSA-375165), and phase 2-plateau phase (REAC: R-HSA-5576893) in Families 1 and 4, and interaction between L1 and Ankyrins (REAC: R-HSA-445095) in Family 3.

The article "Integrative Functional Genomic Analysis in Multiplex Autism Families from Kazakhstan" was published in 2022. Journal: Dis Markers.

## 4. Discussion

Recent studies suggest that in models of the genetic architecture of ASD, common and rare variants interact additively to form susceptibility [47–49]. Common variants likely play a major role in population-level susceptibility, whereas rare mutations contribute substantially to individual susceptibility [21]. Following this hybrid model, we used polygenic risk scores to analyze four extended pedigrees of Kazakhstani ancestry and prioritized ASD risk genes with common and rare inherited and DNM variants. The combination of ASD and BAP was used to improve the performance of risk gene identification. We then performed integrative analysis by constructing PPI networks. We were particularly interested in the nodal elements of the obtained PPI networks. We hypothesized that any perturbation at these important nodes could trigger abnormal conditions such as diseases [50, 51]. According to the obtained results, ten genes clearly formed potentially important nodes in the PPI networks. Six of these genes, namely HDAC4, MECP2, TCF4, TRIM33, TTN, and TSC2, belong to the SFARI category 1-2 (high-confidence and strong candidate genes) and are widely associated with the neuropathological mechanisms of ASD [31, 52–70]. The CFTR, NOD2, PPP2R2B, and TTR genes were not found in the SFARI databases, and data on the role of these genes in ASD are very sparse [71, 72]. However, although the exact mechanism is not clear, there is some evidence of a link between these genes and ASD. The CFTR gene controls secretion and absorption of ions and water in epithelial tissues [73]. Immunohistochemical staining with a mouse monoclonal antibody directed against the C-terminal amino acid sequence of human CFTR revealed diffuse neuronal expression of CFTR in ten human control fetuses at 13 to 40 weeks of gestation [74]. This study showed that CFTR has an early and widespread distribution during development. In addition, a case of autism associated with a genetic variant of CFTR and early exposure to herpes simplex virus (HSV) has been described [71]. The NOD2 gene belongs to the intracellular NOD-like receptor family and plays an important role in the immune response to intracellular bacterial lipopolysaccharides (LPS) [75]. The central role in maintaining the balance between the gut microbiota and the host immune response to control inflammation [76] makes NOD2 one of the most important susceptibility genes for inflammatory bowel diseases [77–82]. At the same time, a number of studies confirm that autistic children are at higher risk for this disorder [83–88]. Moreover, there is evidence of an association between maternal inflammatory bowel disease and ASD in children [89, 90]. The PPP2R2B gene encodes a neuron-specific B regulatory subunit of protein phosphatase 2 (PP2A), which regulates synaptic plasticity [91]. Some studies suggested that DNMs in the PPP2R2B gene may partially contribute to the genetic landscape of intellectual disability [92], but we found only one study linking this gene to ASD [72]. However, this gene may be a strong ASD candidate given a recent study, which highlights a role of another subunit of PP2A (PPP2R5D) in dendrites and synapses using neuron-specific protein network of ASD risk genes [31]. Another strong candidate may be the TTR gene, which is involved in the transport of thyroid [93] and retinol [94]. The involvement of TTR in novel functions, such as neuroprotection, is part of the very recent and constantly evolving knowledge [95]. In addition, TTR has been shown to interact with the GABA_A_ receptor subunit and regulate its expression and function [96]. GABA receptors play an important role in brain development and synchronization of neural network activity. Since these receptors are located on synaptic and extrasynaptic membranes, a deficiency of GABA receptors leads to a lack of neurotransmission and is associated with ASD [97, 98]. Considering that disease genes tend to cluster and cooccur at central sites in the network [48], the above-mentioned genes may represent a priority list for further validation studies.

The article "Integrative Functional Genomic Analysis in Multiplex Autism Families from Kazakhstan" was published in 2022. Journal: Dis Markers.

Another rationale for constructing a PPI network with ASD and BAP risk genes was to identify convergent signaling pathways. Despite the multiplicity of ASD risk genes in each pedigree, our results suggest overlapping functions involving a limited number of biological pathways. Thus, most of the ASD networks is localized in specific cellular compartments such as axons, ion channel complex, and synapses, whereas most biological processes involve ion channel activity, regulation of synaptic function, and membrane depolarization. These findings confirm the results of previous studies that described synaptic functions and ion channel activity in the development of ASD [31, 99–102] and allow us to hypothesize that the main course of development of autistic traits from BAP to ASD does not change. However, we also identified several novel or poorly characterized signaling pathways, such as circadian entrainment, neural cell adhesion molecule 1 (NCAM1) interaction, butyrophilin family (BTN2 and BTN3) interaction, and the interaction between L1 and ankyrins. The first of these pathways may be of particular interest given the growing evidence for circadian disruption in ASD patients [103–105]. The genes that form NCAM1 interactions gene set are involved in neuronal development and synaptic plasticity [106], and perhaps this pathway is not so unexpected for ASD. Apparently, NCAM1 can be considered a general vulnerability factor for neurological and psychiatric disorders [107]. The role of BTN2 and BTN3 and related proteins in the neurodevelopmental disorders is much less studied [108, 109]. BTNs are regulators of immune responses and exert both stimulatory and inhibitory effects on immune cells [110–112]. The BTN enriched gene set correlates a previous finding of a dysregulated immune system in ASD [113–120]. Ankyrin B (AnkB) is an adaptor and scaffold for motor proteins and various ion channels that is expressed ubiquitously in the organism, including the brain [121]. L1 interaction with AnkB mediates branching and synaptogenesis of cortical inhibitory neurons. AnkB mutations and polymorphisms are associated with ASD [23, 69, 122, 123], but the detailed mechanisms underlying the neurological symptoms associated with AnkB are unknown. Interestingly, both the NCAM1 interaction pathway and the interaction between L1 and ankyrins were prioritized in a study of the role of rare variants in biological processes and molecular pathways leading to the pathogenesis of Alzheimer's disease [124], indicating the prospects for their further investigation in the context of neurological disorders.

The article "Integrative Functional Genomic Analysis in Multiplex Autism Families from Kazakhstan" was published in 2022. Journal: Dis Markers.

The final important finding of our study is the identification of DNMs in affected children. Detailed information on these DNMs can be found in Table 6. Some of these DNMs have been previously described in ASD and/or other neurodevelopmental disorders [125–130], and others are indirectly associated with ASD. In this context, the p.Ala797Asp mutation in the potassium channel gene KCNH2 was of particular interest. This DNM results in a nonconservative amino acid exchange of a nonpolar alanine residue for a negatively charged aspartic acid residue at a conservative position (https://www.ncbi.nlm.nih.gov/clinvar/variation/200440/). An *in silico* analysis revealed that this mutation affects the protein structure or functions (https://www.ncbi.nlm.nih.gov/clinvar/variation/200440/). The data on the clinical significance of this variant are lacking. This study appears to be the first report on this DNM in an affected individual.

Taken together, the DNMs that we found only in children with ASD cannot explain the heritable nature of ASD in the studied families. However, because their greatest number was found in children with severe autism (child AU209 with the most severe ASD has four DNMs), we can assume that dbSNP and rare inherited variants represent a common genomic burden. Their combinations converge in common biological processes and likely contribute to the increased threshold of susceptibility to ASD, while the severity of ASD is determined by DNMs. Similarly, it has been previously reported that patients carrying DNMs in two or more candidate genes exhibit more severe phenotypes of ASD [131]. At the same time, the results showed that the genetic heterogeneity of ASD is so great that different DNMs could be identified even in siblings.

### 4.1. Limitations

We understand that this study has many limitations given the latest genomic technologies, bioinformatics methods, and the large-scale studies [132–134]. However, paradoxically, the large amount of data generated by these studies has raised new challenges and questions, and many more studies and approaches are needed to unravel the complex mechanisms of ASD. In our brief study, we attempted to use a novel approach by constructing PPI networks based on putative causative genes for ASD and BAP. For our study, we chose extended pedigrees, which provided a good opportunity to examine inherited genetic risk factors. We integrated three major genetic components of ASD, and we believe that the genes identified in this study are considered penetrant enough to cause ASD-related traits and should be prioritized for further validation. However, the number of variants that microarrays can contain is limited. GSA tends to focus on relatively common variants, so the study has a bias in its design. It is possible that other undetected or uncharacterized variants not included in this study play a critical role. Risk alleles may be at the level of rare inherited copy number variants (CNVs) [135–138]; therefore, examination of CNVs within these families will be a subject of further study. In addition, we performed our analysis with samples that came mainly from families of Kazakh descent. For this reason, our results cannot be generalized to other populations without further investigation. Future approaches should ideally use whole-genome sequencing in extended pedigrees of not only Kazakh ancestry in conjunction with comprehensive clinical validation of detected deleterious variants.

The article "Integrative Functional Genomic Analysis in Multiplex Autism Families from Kazakhstan" was published in 2022. Journal: Dis Markers.

## 5. Conclusion

This study is an attempt to describe the genetic trajectory of autistic trait development in four extended pedigrees of Kazakhstani ancestry. Construction of networks based on putative causative genes for ASD and BAP revealed no differences in major functional pathways compared with those shown in previous studies for ASD only. Nevertheless, our study uncovered several nodal genes and signaling pathways that have not previously been associated with ASD but for whose relevance there are strong biological arguments. The obtained results highlight the importance of including subclinical phenotypes in the search for inherited causes of ASD and provide insights into previously unknown convergent disease pathways. The study is also interesting regarding new DNMs that may contribute to the pathogenesis of ASD.

## Figures and Tables

**Figure 1:** Family trees. Filled symbols indicate children with ASD, and half-filled symbols indicate BAP carriers. Information on year of birth, nationality, and CARS or BAPQ score is presented for each individual.

**Figure 2:** PPI networks for four families visualized by OmicsNet 2.0. The size of the modules is proportional to their degree.

**Table 1:** Characteristics of dbSNPs, associated with ASD according to the GWAS database.

No.	Region	Mapped_gene	SNP	Context	Risk allele frequency	Family no
1		TRIM33	rs6537825	missense_variant	*A* = 0.085217 (31257/366794, ALFA) *A* = 0.092924 (24596/264690, TOPMED) *A* = 0.115222 (28970/251428, GnomAD_exome)	2; 3; 4
2		AMPD1	rs926938	intergenic_variant	*A* = 0.474113 (125493/264690, TOPMED) *A* = 0.499930 (114386/228804, ALFA) *A* = 0.480234 (67204/139940, GnomAD)	1; 2; 3; 4
3	12q23.1	Y_RNA-NA	rs6538761	intron_variant	*A* = 0.349973 (99039/282990, ALFA) *A* = 0.339321 (89815/264690, TOPMED) *A* = 0.332810 (46600/140020, GnomAD)	1; 2; 3; 4
4			rs4307059	intron_variant	*C* = 0.354951/79164 (ALFA)	1; 2; 3; 4
5	8q24.13	SMILR	rs12543592	intron_variant	*G* = 0.450958 (67558/149810, ALFA)	1; 2; 3; 4
6	17p13.3	SGSM2	rs2447097	intron_variant	*T* = 0.421255 (111502/264690, TOPMED) *T* = 0.457423 (72131/157690, ALFA) *T* = 0.422399 (59146/140024, GnomAD)	1; 2; 3; 4
7	1p21.1	NA-CDK4P1	rs11184553	intergenic_variant	*A* = 0.487925 (129149/264690, TOPMED) *A* = 0.43423 (13263/30544, ALFA)	2; 3; 4
8	5q21.2	LOC105379109	rs325485	intron_variant	*A* = 0.336235 (88998/264690, TOPMED) *A* = 0.383385 (96695/252214, ALFA) *A* = 0.343482 (48025/139818, GnomAD)	1
9	6p22.1	GPR89P-RSL24D1P1	rs17693963	intergenic_variant	*C* = 0.07605 (6941/91270, ALFA)	4
10	10q25.1	SORCS3	rs1021363	intron_variant	*A* = 0.253202 (67020/264690, TOPMED) *A* = 0.261206 (36609/140154, GnomAD) *A* = 0.30279 (6616/21850, ALFA)	1; 2; 3; 4
11	14q32.33	RNU7-160P, BAG5	rs10149470	regulatory_region_variant	*A* = 0.453024 (119911/264690, TOPMED) *A* = 0.450706 (63125/140058, GnomAD) *A* = 0.47706 (22524/47214, ALFA)	1; 2; 3; 4
12	1p31.1	NEGR1	rs1620977	intron_variant	*A* = 0.201863 (53431/264690, TOPMED) *A* = 0.267664 (59447/222096, ALFA) *A* = 0.204083 (28452/139414, GnomAD)	1; 3; 4
13	3p14.2	CADPS	rs1452075	intron_variant	*C* = 0.275542 (85602/310668, ALFA) *C* = 0.263913 (69855/264690, TOPMED) *C* = 0.264183 (37011/140096, GnomAD)	1; 2; 3
14	5q33.2	GALNT10	rs34509057	intron_variant	*A* = 0.165276 (43747/264690, TOPMED) *A* = 0.178673 (25035/140116, GnomAD) *A* = 0.20461 (5869/28684, ALFA)	1
15	11q24.2	NRGN	rs55661361	intron_variant	*A* = 0.434229 (114936/264690, TOPMED) *A* = 0.436872 (61128/139922, GnomAD) *A* = 0.29541 (7146/24190, ALFA)	1; 2; 3; 4
16	2p16.1	ACTG1P22	rs11682175	intron_variant	*C* = 0.378579 (100206/264690, TOPMED) *C* = 0.381349 (53401/140032, GnomAD) *C* = 0.44219 (37947/85816, ALFA)	1; 2; 3
17	Xp22.12	LOC105373146	rs1378559	intron_variant	*C* = 0.102214 (27055/264690, TOPMED) *C* = 0.103850 (10650/102552, GnomAD) *C* = 0.13327 (4653/34914, ALFA)	2; 4
18	7q21.11	PCLO	rs2522831	intron_variant	*C* = 0.420114 (111200/264690, TOPMED) *C* = 0.451828 (70140/155236, ALFA) *C* = 0.412847 (57811/140030, GnomAD)	1; 2; 3; 4
19	18q21.2	DCC	rs10164055	intron_variant	*C* = 0.292176 (77336/264690, TOPMED) *C* = 0.316869 (44375/140042, GnomAD)	1
20	18q21.2	TCF4	rs12967143	intron_variant	*G* = 0.475005 (125729/264690, TOPMED) *G* = 0.453865 (63532/139980, GnomAD)	1; 2; 3; 4
21	20q13.12	SLC12A5	rs12624433	intron_variant	*A* = 0.196184 (51928/264690, TOPMED) *A* = 0.202170 (28328/140120, GnomAD) *A* = 0.18751 (6001/32004, ALFA)	1; 2; 4
22	18q21.2	NA-LINC01929	rs11874716	intergenic_variant	*G* = 0.397461 (105204/264690, TOPMED) *G* = 0.33788 (10187/30150, ALFA)	2; 4
23		LINC02551	rs10791097	intron_variant	*T* = 0.396830 (105037/264690, TOPMED) *T* = 0.404173 (56615/140076, GnomAD) *T* = 0.42591 (10204/23958, ALFA)	1; 2; 3; 4
24	3p14.2	FHIT	rs1353545	intron_variant	*C* = 0.377823 (100006/264690, TOPMED) *C* = 0.359634 (50292/139842, GnomAD) *C* = 0.35375 (7099/20068, ALFA)	1; 2; 3
25	3p22.2	HSPD1P6-LINC02033	rs75968099	intergenic_variant	*T* = 0.250519 (66310/264690, TOPMED) *T* = 0.259647 (36321/139886, GnomAD) *T* = 0.31905 (11244/35242, ALFA)	1; 3
26	11q24.1	GRAMD1B	rs77502336	intron_variant	*C* = 0.271272 (71803/264690, TOPMED) *C* = 0.270710 (37940/140150, GnomAD) *C* = 0.28936 (5315/18368, ALFA)	2; 3; 4
27	5q31.2	ETF1	rs3849046	intron_variant	*C* = 0.492134 (130263/264690, TOPMED) *C* = 0.49090 (37400/76186, ALFA)	1; 2; 3; 4
28	14q24.2	RGS6	rs2332700	intron_variant	*C* = 0.237391 (62835/264690, TOPMED) *C* = 0.240436 (33662/140004, GnomAD) *C* = 0.25146 (4750/18890, ALFA)	1; 2; 3; 4
29	12p13.33	CACNA1C	rs1024582	intron_variant	*A* = 0.235419 (62313/264690, TOPMED) *A* = 0.300859 (31805/105714, ALFA)	1; 2; 4
30	4q33	CLCN3	rs10520163	intron_variant	*C* = 0.499018 (175400/351490, ALFA) *C* = 0.442945 (117243/264690, TOPMED) *C* = 0.440639 (61678/139974, GnomAD)	1; 2; 3; 4
31	7q33	DGKI	rs3735025	3_prime_UTR_variant	*C* = 0.288232 (76292/264690, TOPMED) *C* = 0.286664 (40102/139892, GnomAD) *C* = 0.33618 (19781/58840, ALFA)	1; 2; 3; 4
32	5q12.1	SMIM15-AS1	rs171748	intron_variant	*A* = 0.389289 (103041/264690, TOPMED) *A* = 0.395943 (55421/139972, GnomAD)	1; 2; 3; 4
33	17p13.3	SRR	rs4523957	intron_variant	*G* = 0.460962 (122012/264690, TOPMED) *G* = 0.456330 (63899/140028, GnomAD) *G* = 0.40695 (13754/33798, ALFA)	3; 4
34	6p22.2	BTN2A1	rs1977199	intron_variant	*G* = 0.335797 (88882/264690, TOPMED) *G* = 0.332093 (46319/139476, GnomAD)	1; 2; 3; 4
35		TSNARE1	rs4129585	intron_variant	*A* = 0.312399 (82689/264690, TOPMED) *A* = 0.415568 (85636/206070, ALFA) *A* = 0.327265 (45819/140006, GnomAD)	1; 2; 3; 4
36	14q32.33	COA8	rs12887734	intron_variant	*T* = 0.248290 (65720/264690, TOPMED) *T* = 0.258449 (35666/138000, GnomAD) *T* = 0.27298 (5156/18888, ALFA)	1; 2; 3; 4
37	5q33.2	GRIA1	rs12522290	regulatory_region_variant	*G* = 0.115290 (30516/264690, TOPMED) *G* = 0.121303 (17003/140170, GnomAD) *G* = 0.14219 (2686/18890, ALFA)	4
38	6p21.1	ZNF318	rs73416724	non_coding_transcript_exon_variant	*G* = 0.108221 (28645/264690, TOPMED) *G* = 0.106380 (14899/140054, GnomAD) *G* = 0.11175 (2111/18890, ALFA)	1
39		CACNB2	rs7893279	intron_variant	*G* = 0.102354 (27092/264690, TOPMED) *G* = 0.102536 (14367/140116, GnomAD) *G* = 0.11104 (8492/76480, ALFA)	1; 3; 4
40	6p21.33	MSH5, MSH5-SAPCD1	rs707939	intron_variant	*A* = 0.359700 (113481/315488, ALFA) *A* = 0.258582 (68444/264690, TOPMED) *A* = 0.343005 (85522/249332, GnomAD_exome)	1; 2; 3; 4
41	8q24.3	TSNARE1	rs67756423	intron_variant	*C* = 0.215191 (56959/264690, TOPMED) *C* = 0.207610 (29092/140128, GnomAD)	2; 4
42		CACNA1I	rs5995756	intron_variant	*T* = 0.401938 (106389/264690, TOPMED) *T* = 0.443669 (63426/142958, ALFA) *T* = 0.383588 (53667/139908, GnomAD)	1; 2; 3; 4
43	6p22.1	MIR3143-RPL10P2	rs911186	intergenic_variant	*G* = 0.254724 (67423/264690, TOPMED) *G* = 0.224222 (37589/167642, ALFA) *G* = 0.247801 (34709/140068, GnomAD)	3; 4
44	15q25.1	CHRNA3	rs8042374	intron_variant	*G* = 0.316495 (83773/264690, TOPMED) *G* = 0.250356 (58410/233308, ALFA) *G* = 0.286205 (39794/139040, GnomAD)	1; 2; 3; 4
45	3p26.3	CNTN4	rs17194490	intron_variant	*T* = 0.14142 (11348/80244, ALFA)	3; 4
46	6p22.2	BTN3A2	rs13218591	3_prime_UTR_variant	*C* = 0.302939 (80185/264690, TOPMED) *C* = 0.299397 (41927/140038, GnomAD) *C* = 0.30182 (24657/81694, ALFA)	3; 4
47	6p21.33	MUCL3, SFTA2	rs3132581	intron_variant	*A* = 0.089059 (23573/264690, TOPMED) *A* = 0.124702 (20499/164384, ALFA) *A* = 0.094994 (13286/139862, GnomAD)	4
48	2q37.1	SNORC	rs2675968	intron_variant	*T* = 0.301515 (79808/264690, TOPMED) *T* = 0.301837 (42253/139986, GnomAD) *T* = 0.30176 (9576/31734, ALFA)	1; 2
49	10q22.3	ZMIZ1	rs703970	intron_variant	*A* = 0.380653 (100755/264690, TOPMED) *A* = 0.408319 (94164/230614, ALFA) *A* = 0.379565 (53168/140076, GnomAD	2; 3; 4
50	2q32.1	ZNF804A	rs7597593	intron_variant	*T* = 0.475753 (125927/264690, TOPMED) *T* = 0.403458 (85471/211846, ALFA) *T* = 0.470696 (65791/139774, GnomAD)	3; 4
51	7q33	NA-ZP3P2	rs10250997	intergenic_variant	*A* = 0.144509 (38250/264690, TOPMED) *A* = 0.114385 (23197/202798, ALFA) *A* = 0.147202 (20600/139944, GnomAD)	2; 4
52	3p22.2	HSPD1P6, LINC02033	rs9834970	Regulatory region variant	*C* = 0.455287 (120510/264690, TOPMED) *C* = 0.498254 (88177/176972, ALFA) *C* = 0.443239 (62057/140008, GnomAD)	1; 2; 3
53	2p16.3	FOXN2-PPP1R21-DT	rs7565792	intergenic_variant	*T* = 0.433488 (114740/264690, TOPMED) *T* = 0.403518 (63605/157626, ALFA)	1; 2; 4
54	10p14	LOC105376387	rs6602217	intron_variant	*C* = 0.084034 (24182/287766, ALFA) *C* = 0.158298 (41900/264690, TOPMED) *C* = 0.156390 (21899/140028, GnomAD)	3; 4
55	16p13.2	LOC101927026	rs12325410	intron_variant	*G* = 0.156282 (45041/288204, ALFA) *G* = 0.172092 (45551/264690, TOPMED) *G* = 0.163921 (22966/140104, GnomAD)	1; 2; 4
56	16p13.2	GRIN2A	rs8058295	intron_variant	*A* = 0.320919 (84944/264690, TOPMED) *A* = 0.325310 (45557/140042, GnomAD) *A* = 0.28528 (24029/84230, ALFA)	3; 4
57			rs6694545		*A* = 0.268749 (73956/275186, ALFA) *A* = 0.433889 (114846/264690, TOPMED) *A* = 0.417634 (58432/139912, GnomAD)	1; 3; 4
58	8p12	RPL10AP3-NA	rs2609653	intergenic_variant	*C* = 0.054090 (14317/264690, TOPMED) *C* = 0.051313 (12505/243702, ALFA) *C* = 0.059383 (8325/140192, GnomAD)	2; 4
59	18q21.2	RNA5SP459-TCF4	rs9951150	intergenic_variant	*A* = 0.482444 (127698/264690, TOPMED) *G* = 0.456371 (105084/230260, ALFA) *A* = 0.486253 (68018/139882, GnomAD)	1; 2; 3
60	1p31.1	NA-ADGRL4	rs10873998	intergenic_variant	*T* = 0.466702 (112367/240768, ALFA)	1; 2; 3; 4
61	15q25.3	NTRK3	rs1104918	intron_variant	*G* = 0.239850 (63486/264690, TOPMED) *G* = 0.19576 (6837/34926, ALFA)	1; 4
62	2q11.2	IL1R2, IL1R1	rs2310173	intron_variant	*T* = 0.455849 (131145/287694, ALFA) *T* = 0.358208 (94814/264690, TOPMED)	2; 3; 4
63	13q33.3		rs12871532	intergenic_variant	*C* = 0.460323 (121843/264690, TOPMED) *C* = 0.454100 (63544/139934, GnomAD)	1; 2; 3; 4
64	5q32	PPP2R2B	rs609412	intron_variant	*G* = 0.260245 (91536/351730, ALFA) *G* = 0.376361 (99619/264690, TOPMED) *G* = 0.355398 (49770/140040, GnomAD)	1; 2; 3; 4
65	4q31.3	RNA5SP169	rs360932	intron_variant	*G* = 0.443636 (117426/264690, TOPMED) *G* = 0.437177 (61189/139964, GnomAD) *G* = 0.38767 (20945/54028, ALFA)	1; 2; 3; 4
66	2q31.3		rs13418455	intergenic_variant	*T* = 0.342787 (93958/274100, ALFA) *T* = 0.283577 (75060/264690, TOPMED) *T* = 0.293173 (41009/139880, GnomAD)	2; 3; 4
67	2q37.3	HDAC4	rs3791556	intron_variant	*A* = 0.163726 (49335/301326, ALFA) *A* = 0.171291 (45339/264690, TOPMED) *A* = 0.162051 (22715/140172, GnomAD)	1; 2; 3; 4
68	1p31.1		rs4650608	intergenic_variant	*C* = 0.280812 (74328/264690, TOPMED) *C* = 0.312248 (56703/181596, ALFA) *C* = 0.293815 (41147/140044, GnomAD)	4
69	7p22.3	MRM2	rs7799006	3_prime_UTR_variant	*T* = 0.353602 (101853/288044, ALFA) *T* = 0.344482 (91181/264690, TOPMED) *T* = 0.333479 (46647/139880, GnomAD)	1; 2; 3
70	8p12	PPP1R3B, RPL10AP3	rs6990255	intron_variant	*T* = 0.048947 (15545/317586, ALFA) *T* = 0.100899 (26707/264690, TOPMED) *T* = 0.103487 (14494/140056, GnomAD)	2; 4
71	9p24.3	SMARCA2-RN7SL592P	rs4741652	intergenic_variant	*C* = 0.218916 (57945/264690, TOPMED) *C* = 0.266060 (50818/191002, ALFA)	1; 2; 3; 4
72	10q21.2	ANK3	rs10994359	intron_variant	*C* = 0.086131 (22798/264690, TOPMED) *C* = 0.077921 (10922/140168, GnomAD)	1; 2; 3; 4

The article "Integrative Functional Genomic Analysis in Multiplex Autism Families from Kazakhstan" was published in 2022. Journal: Dis Markers.

**Table 2:** Characteristics of rare inherited variants.

No.	Name	SIFT/PolyPhen	Clinical significance (last reviewed)	dbSNP ID	GMAF	Type	Family No.
1	NM_000055.2 (BCHE):c.293A>G (p.Asp98Gly)	Deleterious (0.01)/possibly damaging (0.511)	Pathogenic/likely pathogenic (last reviewed: May 29, 2020)	rs1799807	0.00599 (C)	Missense variant	1
2	NM_019000.4 (RETREG1):c.503C>G (p.Ser168Ter)	-/-	Pathogenic (last reviewed: Jun 3, 2020)	rs137852739	0.00020 (A)	Stop gained	1; 2; 3; 4
3	NM_004646.3 (NPHS1):c.2869G>A (p.Val957Met)	Deleterious (0.02)/probably damaging (0.995)	Likely pathogenic (last reviewed: May 25, 2018)	rs114849139	0.00280 (G)	Missense variant	2
4	NM_017882.3 (CLN6):c.307C>T (p.Arg103Trp)	Deleterious (0)/probably damaging (0.999)	Conflicting interpretations of pathogenicity (last reviewed: Sep 21, 2020)	rs201095412	0.00020 (A)	Missense variant	4
5	NM_000256.3 (MYBPC3):c.649A>G (p.Ser217Gly)	Deleterious (0.01)/possibly damaging (0.541)	Conflicting interpretations of pathogenicity (last reviewed: Sep 20, 2021)	rs138753870	0.00180 (C)	Missense variant	4
6	NM_000369.5 (TSHR):c.1349G>A (p.Arg450His)	Deleterious (0)/probably damaging (0.999)	Conflicting interpretations of pathogenicity (last reviewed: Sep 1, 2021)	rs189261858	0.00020 (A)	Missense variant	4
7	NM_003122.4 (SPINK1):c.194+2T>C	-/-	Conflicting interpretations of pathogenicity (last reviewed: Oct 7, 2020)	rs148954387	0.00080 (G)	Splice donor variant	3
8	NM_000036.3 (AMPD1):c.860A>T (p.Lys287Ile)	Deleterious (0)/probably damaging (1)	Conflicting interpretations of pathogenicity (last reviewed: Oct 31, 2018)	rs34526199	0.01098 (A)	Missense variant	1; 4
9	NM_020631.5 (PLEKHG5):c.2485G>T (p.Asp829Tyr)	Deleterious (0)/possibly damaging (0.876)	Conflicting interpretations of pathogenicity (last reviewed: Oct 29, 2020)	rs200162521	0.00020 (A)	Missense variant	1
10	NM_000540.3 (RYR1):c.9713A>G (p.Glu3238Gly)	Deleterious (0.01)/possibly damaging (0.503)	Conflicting interpretations of pathogenicity (last reviewed: Nov 3, 2020)	rs200950673	0.00020 (G)	Missense variant	4
11	NM_001849.4 (COL6A2):c.2795C>T	Tolerated (0.23)/benign (0.041)	Conflicting interpretations of pathogenicity (last reviewed: Nov 27, 2020)	rs117725825	0.00160 (T)	Missense variant	4
12	NM_000335.5 (SCN5A):c.4821C>T (p.Leu1607=)	-/-	Conflicting interpretations of pathogenicity (last reviewed: Nov 25, 2020)	rs45437099	0.00100 (A)	Synonymous variant	3; 4
13	NM_001267550.2(TTN):c.102595A>G (p.Ile34199Val)	-/benign (0.151)	Conflicting interpretations of pathogenicity (last reviewed: Nov 21, 2020)	rs56347248	0.00599 (C)	Missense variant	3
14	NM_001267550.2(TTN):c.101891G>A (p.Arg33964His)	-/benign (0.018)	Conflicting interpretations of pathogenicity (last reviewed: Nov 21, 2020)	rs55669553	0.00599 (T)	Missense variant	3
15	NM_001267550.2(TTN):c.95297C>T (p.Ser31766Phe)	-/probably damaging (0.998)	Conflicting interpretations of pathogenicity (last reviewed: Nov 21, 2020)	rs191484894	0.00599 (A)	Missense variant	3
16	NM_001267550.2(TTN):c.90536G>A (p.Arg30179His)	-/probably damaging (0.998)	Conflicting interpretations of pathogenicity (last reviewed: Nov 21, 2020)	rs149567378	0.00619 (T)	Missense variant	3
17	NM_001267550.2(TTN):c.82560C>A (p.Asn27520Lys)	-/probably damaging (0.997)	Conflicting interpretations of pathogenicity (last reviewed: Nov 21, 2020)	rs56264840	0.00579 (T)	Missense variant	3
18	NM_001267550.2(TTN):c.49919G>C (p.Ser16640Thr)	-/probably damaging (0.991)	Conflicting interpretations of pathogenicity (last reviewed: Nov 21, 2020)	rs55663050	0.00599 (G)	Missense variant	3
19	NM_001267550.2(TTN):c.47545C>A (p.Pro15849Thr)	-/benign (0.15)	Conflicting interpretations of pathogenicity (last reviewed: Nov 21, 2020)	rs146181477	0.00599 (T)	Missense variant	3
20	NM_001267550.2(TTN):c.1137A>G (p.Arg379=)	-/-	Conflicting interpretations of pathogenicity (last reviewed: Nov 21, 2020)	rs55972547	0.00599 (C)	Synonymous variant	3
21	NM_172364.5(CACNA2D4):c.2120G>A (p.Arg707His)	Tolerated (0.4)/possibly damaging (0.795)	Conflicting interpretations of pathogenicity (last reviewed: Nov 18, 2020)	rs76064926	0.00719 (T)	Missense variant	3
22	NM_018100.4(EFHC1):c.685T>C (p.Phe229Leu)	Tolerated (0.12)/benign (0.039)	Conflicting interpretations of pathogenicity (last reviewed: May 5, 2021)	rs137852776	0.00180 (C)	Missense variant	3
23	NM_003126.4(SPTA1):c.6421C>T (p.Arg2141Trp)	Deleterious (0.01)/probably damaging (1)	Conflicting interpretations of pathogenicity (last reviewed: May 30, 2019)	rs41273519	0.00160 (A)	Missense variant	4
24	NM_001271208.2(NEB):c.571G>C (p.Glu191Gln)	Deleterious (0.09)/probably damaging (0.999)	Conflicting interpretations of pathogenicity (last reviewed: May 18, 2021)	rs35686968	0.00719 (G)	Missense variant	3
25	NM_000784.4(CYP27A1):c.1151C>T (p.Pro384Leu)	Deleterious (0)/probably damaging (0.991)	Conflicting interpretations of pathogenicity (last reviewed: May 18, 2021)	rs41272687	0.00859 (T)	Missense variant	3
26	NM_000237.3(LPL):c.953A>G (p.Asn318Ser)	Tolerated (0.24)/benign (0.137)	Conflicting interpretations of pathogenicity (last reviewed: May 18, 2021)	rs268	0.00519 (G)	Missense variant	1
27	NM_000243.2(MEFV):c.1772T>C (p.Ile591Thr)	Tolerated (0.55)/benign (0)	Conflicting interpretations of pathogenicity (last reviewed: May 18, 2021)	rs11466045	0.00439 (G)	Missense variant	1
28	NM_001370466.1(NOD2):c.332G>A (p.Arg111Gln)	Deleterious (0)/benign (0.116)	Conflicting interpretations of pathogenicity (last reviewed: May 14, 2018)	rs104895456	0.00020 (A)	Missense variant	4
29	NM_014588.5(VSX1):c.479G>A (p.Gly160Asp)	Tolerated (0.3)/benign (0.156)	Conflicting interpretations of pathogenicity (last reviewed: Mar 6, 2018)	rs74315433	0.00260 (A)	Missense variant	4
30	NM_020812.4(DOCK6):c.4862T>C (p.Val1621Ala)	Deleterious (0)/benign (0.161)	Conflicting interpretations of pathogenicity (last reviewed: Mar 19, 2021)	rs201738818	0.00120 (G)	Missense variant	2
31	NM_000136.3(FANCC):c.77C>T (p.Ser26Phe)	Deleterious (0)/probably damaging (0.948)	Conflicting interpretations of pathogenicity (last reviewed: Jun 1, 2021)	rs1800361	0.00260 (A)	Missense variant	2
32	NM_006432.4(NPC2):c.441+1G>A	-/-	Conflicting interpretations of pathogenicity (last reviewed: Jun 1, 2021)	rs140130028	0.00100 (T)	Splice donor variant	3; 4
33	NM_000492.4(CFTR):c.1584G>A (p.Glu528=)	-/-	Conflicting interpretations of pathogenicity (last reviewed: Jul 22, 2021)	rs1800095	0.01058 (A)	Synonymous variant	4
34	NM_001267550.2(TTN):c.14698G>A (p.Ala4900Thr)	-/probably damaging (0.926)	Conflicting interpretations of pathogenicity (last reviewed: Jul 1, 2021)	rs72648923	0.00180 (T)	Missense variant	2
35	NM_001079802.2(FKTN):c.1297A>G (p.Thr433Ala)	Tolerated (0.52)/benign (0.005)	Conflicting interpretations of pathogenicity (last reviewed: Jul 1, 2021)	rs141918432	0.00100 (G)	Missense variant	4
36	NM_022168.4(IFIH1):c.1879G>T (p.Glu627Ter)	-/-	Conflicting interpretations of pathogenicity (last reviewed: Jan 1, 2021)	rs35744605	0.00140 (A)	Stop gained	1
37	NM_001267550.2(TTN):c.48727C>T (p.Pro16243Ser)	-/benign (0.068)	Conflicting interpretations of pathogenicity (last reviewed: Feb 4, 2021)	rs72677242	0.00160 (A)	Missense variant	2
38	NM_000548.5(TSC2):c.1939G>A (p.Asp647Asn)	Deleterious (0.01)/probably damaging (0.995)	Conflicting interpretations of pathogenicity (last reviewed: Dec 7, 2020)	rs45509392	0.00040 (A)	Missense variant	2
39	NM_000371.4(TTR):c.417G>A (p.Thr139=)	-/-	Conflicting interpretations of pathogenicity (last reviewed: Dec 7, 2020)	rs2276382	0.00359 (A)	Synonymous variant	1
40	NM_001267550.2(TTN):c.65775C>T (p.Ser21925=)	-/-	Conflicting interpretations of pathogenicity (last reviewed: Dec 6, 2020)	rs72646867	0.00160 (A)	Synonymous variant	2
41	NM_000527.5(LDLR):c.148G>T (p.Ala50Ser)	Tolerated (0.33)/benign (0.169)	Conflicting interpretations of pathogenicity (last reviewed: Dec 6, 2020)	rs137853960	0.00060 (A)	Missense variant	1
42	NM_012472.6(DNAAF11):c.1391C>T (p.Pro464Leu)	Deleterious (0)/probably damaging [1]	Conflicting interpretations of pathogenicity (last reviewed: Dec 31, 2019)	rs139131485	0.00080 (A)	Missense variant	1
43	NM_005634.2(SOX3):c.157G>C (p.Val53Leu)	Tolerated (0.11)/benign (0.001)	Conflicting interpretations of pathogenicity (last reviewed: Dec 31, 2019)	rs200361128	0.00265 (G)	Missense variant	4
44	NM_000065.4(C6):c.2381+2T>C	-/-	Conflicting interpretations of pathogenicity (last reviewed: Dec 22, 2017)	rs76202909	0.00120 (G)	Splice donor variant	1
45	NM_001037.5(SCN1B):c.28G>A (p.Gly10Ser)	Tolerated (0.4)/possibly damaging (0.862)	Conflicting interpretations of pathogenicity (last reviewed: Dec 2, 2020)	rs72552027	0.00319 (A)	Missense variant	2
46	NM_006214.4(PHYH):c.734G>A (p.Arg245Gln)	Deleterious (0.01)/benign (0.393)	Conflicting interpretations of pathogenicity (last reviewed: Aug 6, 2020)	rs62619919	0.00539 (T)	Missense variant	4
47	NM_201596.3(CACNB2):c.1816C>T (p.Arg606Trp)	Deleterious (0.03)/probably damaging (0.928)	Conflicting interpretations of pathogenicity (last reviewed: Aug 6, 2020)	rs61733968	0.00439 (G)	Missense variant	4
48	NM_000275.3(OCA2):c.1441G>A (p.Ala481Thr)	Tolerated (0.09)/possibly damaging (0.621)	Conflicting interpretations of pathogenicity (last reviewed: Apr 20, 2021)	rs74653330	0.00799 (T)	Missense variant	1;3
49	NM_025216.3(WNT10A):c.511C>T (p.Arg171Cys)	Deleterious (0)/probably damaging (0.93)	Conflicting interpretations of pathogenicity (last reviewed: Apr 13, 2021)	rs116998555	0.00319 (T)	Missense variant	1; 2;3; 4
50	NM_001110792.2(MECP2):c.638C>T (p.Ala213Val)	Tolerated (0.07)/benign (0)	Benign/likely benign (last reviewed: Dec 31, 2019)	rs61748381	0.00477 (A)	Missense variant	4

The article "Integrative Functional Genomic Analysis in Multiplex Autism Families from Kazakhstan" was published in 2022. Journal: Dis Markers.

**Table 3:** DNMs in children with ASD.

Child	Family No.	Name	Clinical significance (last reviewed) ClinVar	Type	dbSNP ID	GMAF
AU 53	1	NM_000162.5(GCK):c.1018A>G (p.Ser340Gly)	Likely pathogenic (last reviewed: Aug 18, 2011)	Missense variant	rs193922255	NA
AU 54	1	NM_138413.4(HOGA1):c.769T>G (p.Cys257Gly)	Pathogenic/likely pathogenic (last reviewed: Sep 21, 2020)	Missense variant	rs267606764	1000 genomes project 0.00020
AU 209	2	NM_000090.3(COL3A1):c.637G>A (p.Gly213Ser)	Pathogenic	Missense variant	rs587779557	NA
AU 209	2	NM_003060.4(SLC22A5):c.287G>C (p.Gly96Ala)	Conflicting interpretations of pathogenicity (last reviewed: Dec 6, 2020)	Missense variant	rs377767450	gnomAD 0.00013
AU 209	2	NM_172107.4(KCNQ2):c.2245G>T (p.Glu749Ter)	Pathogenic (last reviewed: Jan 21, 2020)	Stop gained	rs796052658	ALFA (0/10680) 0.00000
AU 209	2	NM_000071.3(CBS):c.457G>A (p.Gly153Arg)	Pathogenic/likely pathogenic (last reviewed: Jul 24, 2019)	Missense variant	rs745704046	gnomAD, exomes 0.00004
AU 210	2	NM_022455.4(NSD1):c.5146+1G>A	Pathogenic/likely pathogenic (last reviewed: Jul 30, 2019)	Splice donor variant	rs587784139	NA
AU 210	2	NM_006031.6(PCNT):c.5767C>T (p.Arg1923Ter)	Pathogenic/likely pathogenic (last reviewed: Feb 12, 2020)	Stop gained	rs119479062	gnomAD, exomes 0.00001
AU 216	4	NM_000090.3(COL3A1):c.2022G>T (p.Lys674Asn)	Pathogenic	Missense variant	rs587779643	NA
AU 216	4	NM_172056.2(KCNH2):c.2390C>A (p.Ala797Asp)	Likely pathogenic (last reviewed: Jun 12, 2013)	Missense variant	rs794728389	NA
AU 216	4	NM_152722.5(HEPACAM):c.740C>T (p.Thr247Ile)	Uncertain significance (last reviewed: Jan 13, 2018)	Missense variant	rs145619784	1000 genomes project 0.00020
AU 217	4	NM_025216.3(WNT10A):c.1087A>C (p.Asn363His)	Conflicting interpretations of pathogenicity (last reviewed: Dec 3, 2020)	Missense variant	rs34972707	NHLBI ESP exome variant 0.00028

The article "Integrative Functional Genomic Analysis in Multiplex Autism Families from Kazakhstan" was published in 2022. Journal: Dis Markers.

**Table 4:** The list of hub genes with the degree values (degree ≥ 50).

Family No.	ID	Gene	DC
1	9759	HDAC4	202
	6925	TCF4	54
	5521	PPP2R2B	51
	7276	TTR	50

2	9759	HDAC4	202
	7273	TTN	104
	51592	TRIM33	73
	7249	TSC2	62
	6925	TCF4	54
	5521	PPP2R2B	51

3	9759	HDAC4	202
	7273	TTN	104
	51592	TRIM33	73
	6925	TCF4	54
	5521	PPP2R2B	51

4	1080	CFTR	222
	9759	HDAC4	202
	51592	TRIM33	73
	4204	MECP2	60
	6925	TCF4	54
	5521	PPP2R2B	51
	64127	NOD2	50

**Table 5:** Top 15 terms in each GO category and results for REACTOME and KEGG.

Family No.	Source	Term_name	Term_id	Adjusted *p*
1	GO:MF	Voltage-gated calcium channel activity involved in AV node cell action potential	GO:0086056	3,329*E*-04
	GO:MF	Voltage-gated calcium channel activity	GO:0005245	8,797*E*-04
	GO:MF	Voltage-gated calcium channel activity involved in cardiac muscle cell action potential	GO:0086007	1,109*E*-03
	GO:MF	Gated channel activity	GO:0022836	1,270*E*-03
	GO:MF	Ion channel activity	GO:0005216	3,921*E*-03
	GO:MF	Voltage-gated ion channel activity	GO:0005244	4,350*E*-03
	GO:MF	Voltage-gated channel activity	GO:0022832	4,434*E*-03
	GO:MF	High-voltage-gated calcium channel activity	GO:0008331	4,982*E*-03
	GO:MF	Channel activity	GO:0015267	6,566*E*-03
	GO:MF	Passive transmembrane transporter activity	GO:0022803	6,631*E*-03
	GO:MF	Calcium channel activity	GO:0005262	1,450*E*-02
	GO:MF	4-Hydroxy-2-oxoglutarate aldolase activity	GO:0008700	1,696*E*-02
	GO:MF	Inorganic cation transmembrane transporter activity	GO:0022890	1,868*E*-02
	GO:MF	Calcium ion transmembrane transporter activity	GO:0015085	2,112*E*-02
	GO:MF	Cation channel activity	GO:0005261	2,351*E*-02
	GO:BP	Membrane depolarization during action potential	GO:0086010	5,793*E*-06
	GO:BP	Membrane depolarization	GO:0051899	1,478*E*-04
	GO:BP	Calcium ion import	GO:0070509	2,539*E*-04
	GO:BP	Membrane depolarization during cardiac muscle cell action potential	GO:0086012	3,450*E*-04
	GO:BP	Regulation of ion transport	GO:0043269	5,961*E*-04
	GO:BP	Regulation of biological quality	GO:0065008	1,127*E*-03
	GO:BP	Anterograde transsynaptic signaling	GO:0098916	1,414*E*-03
	GO:BP	Chemical synaptic transmission	GO:0007268	1,414*E*-03
	GO:BP	Cation transport	GO:0006812	1,458*E*-03
	GO:BP	Action potential	GO:0001508	1,506*E*-03
	GO:BP	Transsynaptic signaling	GO:0099537	1,579*E*-03
	GO:BP	Membrane depolarization during atrial cardiac muscle cell action potential	GO:0098912	1,645*E*-03
	GO:BP	Regulation of neurotransmitter levels	GO:0001505	1,650*E* − 03
	GO:BP	Regulation of membrane potential	GO:0042391	1,682*E* − 03
	GO:BP	Synaptic signaling	GO:0099536	2,185*E* − 03
	GO:CC	Synaptic membrane	GO:0097060	5,243*E* − 05
	GO:CC	Postsynaptic membrane	GO:0045211	6,704*E* − 05
	GO:CC	Postsynapse	GO:0098794	3,189*E* − 04
	GO:CC	Synapse	GO:0045202	3,561*E* − 04
	GO:CC	Voltage-gated calcium channel complex	GO:0005891	4,325*E* − 04
	GO:CC	T-tubule	GO:0030315	8,299*E* − 04
	GO:CC	Neuron projection	GO:0043005	1,019*E* − 03
	GO:CC	Calcium channel complex	GO:0034704	1,957*E* − 03
	GO:CC	Postsynaptic density	GO:0014069	2,909*E* − 03
	GO:CC	Asymmetric synapse	GO:0032279	3,279*E* − 03
	GO:CC	Glutamatergic synapse	GO:0098978	3,547*E* − 03
	GO:CC	Integral component of plasma membrane	GO:0005887	3,884*E* − 03
	GO:CC	L-type voltage-gated calcium channel complex	GO:1990454	4,532*E* − 03
	GO:CC	Postsynaptic specialization	GO:0099572	4,632*E* − 03
	GO:CC	Axon	GO:0030424	5,015*E* − 03
	REAC	NCAM1 interactions	REAC:R-HSA-419037	2,470*E* − 03
	REAC	NCAM signaling for neurite out-growth	REAC:R-HSA-375165	6,919*E* − 03
	REAC	Phase 2-plateau phase	REAC:R-HSA-5576893	2,470*E* − 02
	REAC	Defective GCK causes maturity-onset diabetes of the young 2 (MODY2)	REAC:R-HSA-5619073	3,866*E* − 02

2	GO:MF	Interleukin-1 receptor activity	GO:0004908	1,217*E* − 02
	GO:MF	Interleukin-1 binding	GO:0019966	2,083*E* − 02
	GO:MF	Cation transmembrane transporter activity	GO:0008324	2,968*E* − 02
	GO:MF	Gated channel activity	GO:0022836	3,603*E* − 02
	GO:BP	Ion transmembrane transport	GO:0034220	1,466*E* − 02
	GO:BP	Cation transport	GO:0006812	2,046*E* − 02
	GO:BP	Regulation of reactive oxygen species biosynthetic process	GO:1903426	2,146*E* − 02
	GO:BP	Regulation of transport	GO:0051049	4,096*E* − 02
	GO:BP	Reactive oxygen species biosynthetic process	GO:1903409	4,859*E* − 02
	GO:CC	Node of Ranvier	GO:0033268	9,149*E* − 04
	GO:CC	Axon initial segment	GO:0043194	4,511*E* − 03
	GO:CC	Synapse	GO:0045202	1,322*E* − 02
	GO:CC	Postsynapse	GO:0098794	2,761*E* − 02
	GO:CC	Glutamatergic synapse	GO:0098978	2,787*E* − 02
	GO:CC	Postsynaptic density	GO:0014069	3,305*E* − 02
	GO:CC	Asymmetric synapse	GO:0032279	3,655*E* − 02
	GO:CC	Synaptic membrane	GO:0097060	4,836*E* − 02
	GO:CC	Postsynaptic specialization	GO:0099572	4,886*E* − 02
	REAC	Interaction between L1 and Ankyrins	REAC:R-HSA-445095	4,993*E* − 02

3	GO:MF	Voltage-gated ion channel activity	GO:0005244	2,709*E* − 03
	GO:MF	Voltage-gated channel activity	GO:0022832	2,786*E* − 03
	GO:MF	Gated channel activity	GO:0022836	5,046*E* − 03
	GO:MF	Ion channel activity	GO:0005216	2,213*E* − 02
	GO:MF	Interleukin-1 receptor activity	GO:0004908	3,967*E* − 02
	GO:MF	Channel activity	GO:0015267	4,309*E* − 02
	GO:MF	Cation transmembrane transporter activity	GO:0008324	4,359*E* − 02
	GO:MF	Passive transmembrane transporter activity	GO:0022803	4,364*E* − 02
	GO:MF	Cation channel activity	GO:0005261	4,642*E* − 02
	GO:BP	Membrane depolarization during action potential	GO:0086010	2,140*E* − 03
	GO:BP	Chemical synaptic transmission	GO:0007268	6,930*E* − 03
	GO:BP	Anterograde transsynaptic signaling	GO:0098916	6,930*E* − 03
	GO:BP	Transsynaptic signaling	GO:0099537	7,659*E* − 03
	GO:BP	Synaptic signaling	GO:0099536	1,026*E* − 02
	GO:BP	Membrane depolarization during cardiac muscle cell action potential	GO:0086012	2,544*E* − 02
	GO:BP	Membrane depolarization during atrial cardiac muscle cell action potential	GO:0098912	2,640*E* − 02
	GO:BP	Signal release from synapse	GO:0099643	4,238*E* − 02
	GO:BP	Neurotransmitter secretion	GO:0007269	4,238*E* − 02
	GO:CC	Postsynapse	GO:0098794	1,950*E* − 03
	GO:CC	Glutamatergic synapse	GO:0098978	2,275*E* − 03
	GO:CC	Z disc	GO:0030018	2,747*E* − 03
	GO:CC	I band	GO:0031674	4,378*E* − 03
	GO:CC	Synaptic membrane	GO:0097060	4,834*E* − 03
	GO:CC	Synapse	GO:0045202	5,661*E* − 03
	GO:CC	Postsynaptic membrane	GO:0045211	8,485*E* − 03
	GO:CC	Ion channel complex	GO:0034702	1,235*E* − 02
	GO:CC	Postsynaptic density	GO:0014069	2,124*E* − 02
	GO:CC	Somatodendritic compartment	GO:0036477	2,218*E* − 02
	GO:CC	Asymmetric synapse	GO:0032279	2,351*E* − 02
	GO:CC	Presynapse	GO:0098793	2,828*E* − 02
	GO:CC	Sarcomere	GO:0030017	2,897*E* − 02
	GO:CC	Voltage-gated calcium channel complex	GO:0005891	3,140*E* − 02
	GO:CC	Postsynaptic specialization	GO:0099572	3,151*E* − 02

4	GO:MF	Gated channel activity	GO:0022836	1,641*E* − 07
	GO:MF	Ion channel activity	GO:0005216	1,256*E* − 06
	GO:MF	Channel activity	GO:0015267	3,180*E* − 06
	GO:MF	Passive transmembrane transporter activity	GO:0022803	3,237*E* − 06
	GO:MF	Voltage-gated ion channel activity	GO:0005244	2,328*E* − 05
	GO:MF	Voltage-gated channel activity	GO:0022832	2,418*E* − 05
	GO:MF	Cation channel activity	GO:0005261	9,049*E* − 05
	GO:MF	Inorganic molecular entity transmembrane transporter activity	GO:0015318	1,140*E* − 04
	GO:MF	Inorganic cation transmembrane transporter activity	GO:0022890	2,734*E* − 04
	GO:MF	Ion transmembrane transporter activity	GO:0015075	4,094*E* − 04
	GO:MF	Voltage-gated calcium channel activity involved in AV node cell action potential	GO:0086056	4,671*E* − 04
	GO:MF	Ligand-gated channel activity	GO:0022834	5,175*E* − 04
	GO:MF	Ligand-gated ion channel activity	GO:0015276	5,175*E* − 04
	GO:MF	Voltage-gated cation channel activity	GO:0022843	5,725*E* − 04
	GO:MF	Cation transmembrane transporter activity	GO:0008324	6,190*E* − 04
	GO:BP	Membrane depolarization during action potential	GO:0086010	2,786*E* − 08
	GO:BP	Regulation of membrane potential	GO:0042391	3,523*E* − 08
	GO:BP	Membrane depolarization	GO:0051899	1,673*E* − 06
	GO:BP	Action potential	GO:0001508	3,104*E* − 05
	GO:BP	Membrane depolarization during atrial cardiac muscle cell action potential	GO:0098912	3,486*E* − 05
	GO:BP	Regulation of biological quality	GO:0065008	5,156*E* − 05
	GO:BP	Multicellular organismal signaling	GO:0035637	6,981*E* − 05
	GO:BP	Behavior	GO:0007610	7,368*E* − 05
	GO:BP	Ion transmembrane transport	GO:0034220	1,226*E* − 04
	GO:BP	Cardiac muscle cell action potential	GO:0086001	2,034*E* − 04
	GO:BP	Regulation of ion transport	GO:0043269	2,416*E* − 04
	GO:BP	Membrane depolarization during AV node cell action potential	GO:0086045	3,473*E* − 04
	GO:BP	Regulation of ion transmembrane transport	GO:0034765	4,035*E* − 04
	GO:BP	Cation homeostasis	GO:0055080	4,197*E* − 04
	GO:BP	Membrane depolarization during cardiac muscle cell action potential	GO:0086012	4,806*E* − 04
	GO:CC	Ion channel complex	GO:0034702	5,650*E* − 07
	GO:CC	Transmembrane transporter complex	GO:1902495	4,620*E* − 06
	GO:CC	Transporter complex	GO:1990351	6,231*E* − 06
	GO:CC	Postsynapse	GO:0098794	6,902*E* − 06
	GO:CC	Synaptic membrane	GO:0097060	1,047*E* − 05
	GO:CC	Postsynaptic membrane	GO:0045211	1,501*E* − 05
	GO:CC	Cation channel complex	GO:0034703	1,982*E* − 05
	GO:CC	Neuron projection	GO:0043005	5,502*E* − 05
	GO:CC	Intrinsic component of plasma membrane	GO:0031226	1,206*E* − 04
	GO:CC	Synapse	GO:0045202	2,776*E* − 04
	GO:CC	Sarcolemma	GO:0042383	3,037*E* − 04
	GO:CC	Cell surface	GO:0009986	5,783*E* − 04
	GO:CC	Voltage-gated calcium channel complex	GO:0005891	6,149*E* − 04
	GO:CC	Postsynaptic density	GO:0014069	8,046*E* − 04
	GO:CC	Plasma membrane region	GO:0098590	9,173*E* − 04
	KEGG	Circadian entrainment	KEGG:04713	3,488*E* − 02
	REAC	NCAM1 interactions	REAC:R-HSA-419037	3,277*E* − 06
	REAC	NCAM signaling for neurite out-growth	REAC:R-HSA-375165	1,888*E* − 05
	REAC	Butyrophilin (BTN) family interactions	REAC:R-HSA-8851680	1,215*E* − 02
	REAC	Long-term potentiation	REAC:R-HSA-9620244	1,438*E* − 02
	REAC	Axon guidance	REAC:R-HSA-422475	2,470*E* − 02
	REAC	Nervous system development	REAC:R-HSA-9675108	3,267*E* − 02
	REAC	Phase 2-plateau phase	REAC:R-HSA-5576893	3,338*E* − 02

The article "Integrative Functional Genomic Analysis in Multiplex Autism Families from Kazakhstan" was published in 2022. Journal: Dis Markers.

**Table 6:** Detailed information about DNMs.

DNM	Gene function	Expression	Supporting evidence, ClinVar
c.1018A>G	Glucokinase, phosphorylates glucose to produce glucose-6-phosphate (the first step in most glucose metabolic pathways)	Pancreas and liver	The variant was changed to likely pathogenic upon submission. Other variants in the GCK gene that alter enzyme activity have been associated with various types of diabetes and hyperinsulinemic hypoglycemia [139]. There is a report showing that neonatal hypoglycemia increases the risk of ASD threefold in children born at term [140].
c.769T>G	4-Hydroxy-2-oxoglutarate aldolase 1, catalyzes the final step in the metabolic pathway of hydroxyproline, releasing glyoxylate and pyruvate	Kidney, liver, heart, fat, and brain	The variant results in a nonconservative amino acid change in the encoded protein sequence. Three of five *in silico* tools predicted a deleterious effect of the variant on protein function. The variant was found at a frequency of 6.4*E* − 05 in 249558 control chromosomes, most notably at a frequency of 0.00082 within the East Asian subpopulation in the gnomAD database. This frequency is not higher than the maximum expected for a pathogenic variant in HOGA1 causing primary hyperoxaluria, type III, (0.0015) and does not allow conclusions to be drawn about the significance of the variant. c.769T > G has been reported in the literature in homozygous and compound heterozygous states in several individuals with primary hyperoxaluria, type III [141–144]. These data indicate that the variant is very likely to be associated with disease. At least one publication reports experimental evidence evaluating an impact on protein function and demonstrated that the variant resulted in no measurable activity [145]. Two clinical diagnostic laboratories have submitted clinical-significance assessments for this variant to ClinVar after 2014 and classified the variant as pathogenic/likely pathogenic. There are reports that hyperoxaluria may be involved in the pathogenesis of ASD in children [146, 147].
c.637G>A c.2022G>T	Collagen type III alpha 1 chain, encoding the pro-alpha1 chains of the collagen type III, is found in extensible connective tissues such as skin, lung, uterus, intestine, and the vascular system, often in association with type I collagen	Gall bladder, placenta, and 12 other tissues	The variants are associated with Ehlers-Danlos syndrome, type 4 [148, 149]. Ehlers-Danlos syndrome type 4 shares several similar neurophenotypes with ASD, such as mood disorders, proprioceptive impairments, sensory hyper/hyposensitivities, eating disorders, and suicidality [150].
c.287G > C	Solute carrier family 22 member 5, transporter for organic cations and a sodium-dependent transporter with high affinity for carnitine Potassium voltage-gated channel subfamily Q member 2, integral membrane proteins of potassium channel	Kidney, small intestine and 23 other tissues Brain, adrenal, and testis	The variant results in a nonconservative amino acid change in the major facilitator superfamily domain (IPR020846) of the encoded protein sequence. Five of five *in silico* tools predicted a deleterious effect of the variant on protein function. The variant allele was found at a frequency of 0.00041 in 195700 control chromosomes. This frequency is not significantly higher than would be expected for a pathogenic variant in SLC22A5 causing systemic primary carnitine deficiency (0.00041 vs. 0.0046), which does not allow to conclude the significance of the variant. c.287G > C has been reported in the literature in several individuals with suspected systemic primary carnitine deficiency [151, 152]. These data do not allow any conclusion about variant significance. At least one publication reports experimental evidence indicating that the variant reduced carnitine transport activity to less than 20% of wild-type in vitro [152]. Three clinical diagnostic laboratories have submitted clinical-significance assessments for this variant to ClinVar after 2014 without evidence for independent evaluation. These laboratories cited the variant with conflicting assessments: one laboratory classified the variant likely pathogenic, one laboratory classified the variant as likely benign, and a third laboratory classified the variant as uncertain significance. Based on the evidence outlined above, until additional information becomes available, the variant was classified as VUS-possibly pathogenic. An association between primary carnitine deficiency and ASD has been reported [153, 154]. It is hypothesized that carnitine deficiency in the brain causes nonsyndromal autism with extreme male tendency [155]. The variant is predicted to result in loss of normal protein function due to protein truncation as the last 124 amino acids of the protein are lost.
c.457G>A	Cystathionine beta-synthase, catalyzes the conversion of homocysteine to cystathionine, the first step of the transsulfuration pathway	Liver, brain and 6 other tissues	The variant involves the modification of a conserved nucleotide located within the pyridoxal phosphate-dependent enzyme domain (InterPro). 5/5 *in silico* tools predict a deleterious outcome for this variant. This variant was found in 1/156632 control chromosomes at a frequency of 0.0000064, which does not exceed the estimated maximum expected allele frequency of a pathogenic CBS variant (0.0030414). In addition, functional studies in yeast suggest that the variant may affect protein function [156]. The variant has been reported in a Saudi Arabian family, in which two affected patients with homocystinuria were homozygous for the variant inherited from unaffected heterozygous parents [157]. There are reports that children with classical homocystinuria may have isolated ASD due to cystathionine-*β*-synthase deficiency [158, 159].
c.5146+1G>A	Nuclear receptor binding SET domain protein 1, enhances androgen receptor transactivation	Testis, thyroid and 25 other tissues	The variant affects a donor splice site in intron 14 of the NSD1 gene. It is expected to disrupt RNA splicing and likely results in an absent or disrupted protein product. Donor and acceptor splice site variants generally result in loss of protein function [160], and loss-of-function variants in NSD1 are known to be pathogenic and the major cause of Sotos syndrome [161–163]. One report found several rare variations of the NSD1 gene in individuals with ASD, although the variants were not considered pathogenic [164].
c.5767C>T	Pericentrin, interacts with the microtubule nucleation component gamma-tubulin and is probably important for the normal functioning of centrosomes, the cytoskeleton, and cell cycle progression	Testis, bone marrow and 24 other tissues	The variant has been classified as pathogenic according to ACMG in the context of microcephalic osteodysplastic primordial dwarfism type II. The variant produces a premature translational stop signal (p.Arg1923∗) in the PCNT gene. It is expected to result in absent or impaired protein product. Loss-of-function variants in PCNT are known to be pathogenic [165, 166].
c.2390C>A	Potassium voltage-gated channel subfamily H member 2, encodes a component of a voltage-activated potassium channel found in cardiac muscle, neurons, and microglia	Bone marrow, testis and 14 other tissues	The variant results in a nonconservative amino acid substitution of a nonpolar alanine residue with a negatively charged aspartic acid residue at a position that is conserved across species. In silico analysis predicts Ala797Asp is probably damaging to the protein structure/function. Mutations in nearby residues (Glu788Asp, Glu788Lys, Arg791Trp, Gly800Glu, Gly800Trp) have been reported in association with Long QT syndrome (LQTS), further supporting the functional importance of this region of the protein. Furthermore, the Ala797Asp variant was not observed in approximately 6,500 individuals of European and African American ancestry in the NHLBI exome sequencing project, indicating it is not a common benign variant in these populations. In summary, while Ala797Asp is a good candidate for a disease-causing mutation, with the clinical and molecular information available at this time we cannot unequivocally determine the clinical significance of this variant.
c.740C>T	Hepatic and glial cell adhesion molecule, acts as a homodimer and is involved in cell motility and cell-matrix interactions	Brain, fat and liver	The variant was classified as a variant of unknown significance for megalencephalic leukoencephalopathy with subcortical cysts. Other rare mutations in the HEPACAM gene have been found to cause either macrocephaly and mental retardation with or without autism or benign familial macrocephaly [129].
c.1087A>C	Wnt family member 10A, a member of the WNT gene family, involved in oncogenesis and several developmental processes, including cell fate regulation and cell patterning during embryogenesis	Skin, placenta and 16 other tissues	The variant was not observed in significant frequency in approximately 5300 individuals of European and African American ancestry in the NHLBI exome sequencing project, suggesting that it is not a common benign variant in these populations. The variant is a semiconservative amino acid substitution that may affect secondary protein structure because these residues differ in some properties. This substitution occurs at a position that is conserved across species, and *in silico* analysis predicts that this variant is likely to affect protein structure/function.

The article "Integrative Functional Genomic Analysis in Multiplex Autism Families from Kazakhstan" was published in 2022. Journal: Dis Markers.

## Data Availability

Genomic data have been deposited in a Cloud file storage and are available at https://drive.google.com/drive/folders/1XyIhBp7i8IJJZq7l-aQ3OI0FoNPW1qi6?usp=sharing. The processed data used to support the findings of this study are included in the provided tables.

## References

[1] Pugsley K., Scherer S. W., Bellgrove M. A., Hawi Z. (2022). Environmental exposures associated with elevated risk for autism spectrum disorder may augment the burden of deleterious de novo mutations among probands. *Molecular Psychiatry*.

[2] Hallmayer J., Cleveland S., Torres A. (2011). Genetic heritability and shared environmental factors among twin pairs with autism. *Archives of General Psychiatry*.

[3] Frazier T. W., Thompson L., Youngstrom E. A. (2014). A twin study of heritable and shared environmental contributions to autism. *Journal of Autism and Developmental Disorders*.

[4] Colvert E., Tick B., McEwen F. (2015). Heritability of autism spectrum disorder in a UK population-based twin sample. *JAMA Psychiatry*.

[5] Nordenbæk C., Jørgensen M., Kyvik K. O., Bilenberg N. (2014). A Danish population-based twin study on autism spectrum disorders. *European Child and Adolescent Psychiatry*.

[6] Martens G. J. M., van Loo K. M. J. (2007). Genetic and environmental factors in complex neurodevelopmental disorders. *Current Genomics*.

[7] Ronald A., Hoekstra R. A. (2011). Autism spectrum disorders and autistic traits: a decade of new twin studies. *American Journal of Medical Genetics, Part B: Neuropsychiatric Genetics*.

The article "Integrative Functional Genomic Analysis in Multiplex Autism Families from Kazakhstan" was published in 2022. Journal: Dis Markers.

[8] Abrahams B. S., Geschwind D. H. (2008). Advances in autism genetics: on the threshold of a new neurobiology. *Nature Reviews Genetics*.

[9] Persico A. M., Bourgeron T. (2006). Searching for ways out of the autism maze: genetic, epigenetic and environmental clues. *Trends in Neurosciences*.

[10] Klauck S. M. (2006). Genetics of autism spectrum disorder. *European Journal of Human Genetics*.

[11] Folstein S., Rutter M. (1977). Infantile autism: a genetic study of 21 twin pairs. *Journal of Child Psychology and Psychiatry*.

[12] Richards S., Aziz N., Bale S. (2015). Standards and guidelines for the interpretation of sequence variants: a joint consensus recommendation of the American College of Medical Genetics and Genomics and the Association for Molecular Pathology. *Genetics in Medicine*.

[13] Piven J., Vieland V. J., Parlier M. (2013). A molecular genetic study of autism and related phenotypes in extended pedigrees. *Journal of Neurodevelopmental Disorders*.

[14] Coon H., Villalobos M. E., Robison R. J. (2010). Genome-wide linkage using the social responsiveness scale in Utah autism pedigrees. *Molecular Autism*.

[15] Woodbury-Smith M., Paterson A. D., Thiruvahindrapduram B. (2015). Using extended pedigrees to identify novel autism spectrum disorder (ASD) candidate genes. *Human Genetics*.

[16] Chapman N. H., Nato A. Q., Bernier R. (2015). Whole exome sequencing in extended families with autism spectrum disorder implicates four candidate genes. *Human Genetics*.

[17] Sasson N. J., Lam K. S. L., Parlier M., Daniels J. L., Piven J. (2013). Autism and the broad autism phenotype: familial patterns and intergenerational transmission. *Journal of Neurodevelopmental Disorders*.

[18] Tick B., Bolton P., Happé F., Rutter M., Rijsdijk F. (2016). Heritability of autism spectrum disorders: a meta-analysis of twin studies. *Journal of Child Psychology and Psychiatry and Allied Disciplines*.

[19] Woodbury-Smith M., Paterson A. D., O’Connor I. (2018). A genome-wide linkage study of autism spectrum disorder and the broad autism phenotype in extended pedigrees. *Journal of Neurodevelopmental Disorders*.

[20] Al-Sarraj Y., Al-Dous E., Taha R. Z. (2021). Family-based genome-wide association study of autism spectrum disorder in middle eastern families. *Genes (Basel)*.

[21] Gaugler T., Klei L., Sanders S. J. (2014). Most genetic risk for autism resides with common variation. *Nature Genetics*.

[22] Alonso-Gonzalez A., Rodriguez-Fontenla C., Carracedo A. (2018). De novo mutations (DNMs) in autism spectrum disorder (ASD): Pathway and network analysis. *Frontiers in Genetics*.

The article "Integrative Functional Genomic Analysis in Multiplex Autism Families from Kazakhstan" was published in 2022. Journal: Dis Markers.

[23] Iossifov I., O’roak B. J., Sanders S. J. (2014). The contribution of de novo coding mutations to autism spectrum disorder. *Nature*.

[24] Sanders S. J., Murtha M. T., Gupta A. R. (2012). De novo mutations revealed by whole-exome sequencing are strongly associated with autism. *Nature*.

[25] Caglayan A. O. (2010). Genetic causes of syndromic and non-syndromic autism. *Developmental Medicine and Child Neurology*.

[26] Hormozdiari F., Penn O., Borenstein E., Eichler E. E. (2015). The discovery of integrated gene networks for autism and related disorders. *Genome Research*.

[27] Sakai Y., Shaw C. A., Dawson B. C. (2011). Protein interactome reveals converging molecular pathways among autism disorders. *Science Translational Medicine*.

[28] Pinto D., Delaby E., Merico D. (2014). Convergence of genes and cellular pathways dysregulated in autism spectrum disorders. *American Journal of Human Genetics*.

[29] Wang Y., Kou Y., Meng D. (2020). Network structure analysis identifying key genes of autism and its mechanism. *Computational and Mathematical Methods in Medicine.*.

[30] Gilman S. R., Iossifov I., Levy D., Ronemus M., Wigler M., Vitkup D. (2011). Rare de novo variants associated with autism implicate a large functional network of genes involved in formation and function of synapses. *Neuron*.

[31] Murtaza N., Cheng A. A., Brown C. O. (2022). *Neuron-specific protein network mapping of autism risk genes identifies shared biological mechanisms and disease relevant pathologies*.

[32] Sullivan J. M., de Rubeis S., Schaefer A. (2019). Convergence of spectrums: neuronal gene network states in autism spectrum disorder. *Current Opinion in Neurobiology*.

[33] Jensen R. A. (2013). The background genetic effect of the genes underlying the broad autism phenotype as a unifying feature in gene x gene and gene x environment causal mechanisms in autism. *OA Autism*.

[34] Losh M., Sullivan P. F., Trembath D., Piven J. (2008). Current developments in the genetics of autism: from phenome to genome. *Journal of Neuropathology and Experimental Neurology*.

[35] Vincent J. B., Melmer G., Bolton P. F. (2005). Genetic linkage analysis of the X chromosome in autism, with emphasis on the fragile X region. *Psychiatric Genetics*.

[36] Chen F. S., Johnson S. C. (2012). An oxytocin receptor gene variant predicts attachment anxiety in females and autism-spectrum traits in males. *Social Psychological and Personality Science*.

[37] Freitag C. M. (2007). The genetics of autistic disorders and its clinical relevance: a review of the literature. *Molecular Psychiatry*.

The article "Integrative Functional Genomic Analysis in Multiplex Autism Families from Kazakhstan" was published in 2022. Journal: Dis Markers.

[38] Moon S. J., Hwang J. S., Shin A. L. (2019). Accuracy of the childhood autism rating scale: a systematic review and meta-analysis. *Developmental Medicine and Child Neurology*.

[39] Sasson N. J., KSL L., Childress D., Parlier M., Daniels J. L., Piven J. (2013). The broad autism phenotype questionnaire: prevalence and diagnostic classification. *Autism Research*.

[40] Hurley R. S. E., Losh M., Parlier M., Reznick J. S., Piven J. (2007). The broad autism phenotype questionnaire. *Journal of Autism and Developmental Disorders*.

[41] den Dunnen J. T. (2016). Sequence variant descriptions: HGVS nomenclature and mutalyzer. *Current Protocols in Human Genetics*.

[42] Lynn D. J., Winsor G. L., Chan C. (2008). InnateDB: facilitating systems-level analyses of the mammalian innate immune response. *Molecular Systems Biology*.

[43] Breuer K., Foroushani A. K., Laird M. R. (2013). Innate DB: systems biology of innate immunity and beyond - recent updates and continuing curation. *Nucleic Acids Research*.

[44] Zhou G., Xia J. (2019). Using omics net for network integration and 3D visualization. *Current Protocols in Bioinformatics*.

[45] Ashburner M., Ball C. A., Blake J. A. (2000). Gene ontology: tool for the unification of biology. *Nature Genetics*.

[46] Reimand J., Isserlin R., Voisin V. (2019). Pathway enrichment analysis and visualization of omics data using g:Profiler, GSEA, Cytoscape and Enrichment Map. *Nature Protocols*.

[47] Weiner D. J., Wigdor E. M., Ripke S. (2017). Polygenic transmission disequilibrium confirms that common and rare variation act additively to create risk for autism spectrum disorders. *Nature Genetics*.

[48] Klei L., McClain L. L., Mahjani B. (2021). How rare and common risk variation jointly affect liability for autism spectrum disorder. *Molecular Autism*.

[49] Chaste P., Roeder K., Devlin B. (2017). The Yin and Yang of autism genetics: how rare de novo and common variations affect liability. *Annual Review of Genomics and Human Genetics.*.

[50] Abedi M., Gheisari Y. (2015). Nodes with high centrality in protein interaction networks are responsible for driving signaling pathways in diabetic nephropathy. *Peer J*.

[51] Johnson C. P., Myers S. M., Council on Children with Disabilities (2007). Identification and evaluation of children with autism spectrum disorders. *Pediatrics*.

[52] Smoller J. W., Kendler K., Craddock N. (2013). Identification of risk loci with shared effects on five major psychiatric disorders: a genome-wide analysis. *The Lancet*.

[53] Kim T., Park J. K., Kim H. J., Chung J. H., Kim J. W. (2010). Association of histone deacetylase genes with schizophrenia in Korean population. *Psychiatry Research*.

The article "Integrative Functional Genomic Analysis in Multiplex Autism Families from Kazakhstan" was published in 2022. Journal: Dis Markers.

[54] Fitzgerald T. W., Gerety S. S., Jones W. D. (2015). Large-scale discovery of novel genetic causes of developmental disorders. *Nature*.

[55] Feliciano P., Zhou X., Astrovskaya I. (2019). Exome sequencing of 457 autism families recruited online provides evidence for autism risk genes. *Npj Genomic Medicine*.

[56] Shibayama A., Cook E. H., Feng J. (2004). MECP2 structural and 3′-UTR variants in schizophrenia autism and other psychiatric diseases: a possible association with autism. *American Journal of Medical Genetics Part B: Neuropsychiatric Genetics*.

[57] Mellén M., Ayata P., Dewell S., Kriaucionis S., Heintz N. (2012). MeCP2 binds to 5hmC enriched within active genes and accessible chromatin in the nervous system. *Cell*.

[58] Cohen S., Gabel H. W., Hemberg M. (2011). Genome-wide activity-dependent MeCP2 phosphorylation regulates nervous system development and function. *Neuron*.

[59] Chao H. T., Chen H., Samaco R. C. (2010). Dysfunction in GABA signalling mediates autism-like stereotypies and Rett syndrome phenotypes. *Nature*.

[60] Degano A. L., Pasterkamp R. J., Ronnett G. V. (2009). MeCP2 deficiency disrupts axonal guidance, fasciculation, and targeting by altering Semaphorin 3F function. *Molecular and Cellular Neuroscience*.

[61] Swanberg S. E., Nagarajan R. P., Peddada S., Yasui D. H., Lasalle J. M. (2009). Reciprocal co-regulation of EGR2 and MECP2 is disrupted in Rett syndrome and autism. *Human Molecular Genetics*.

[62] Steinberg S., de Jong S., Andreassen O. A. (2011). Common variants at VRK2 and TCF4 conferring risk of schizophrenia. *Human Molecular Genetics*.

[63] Iossifov I., Levy D., Allen J. (2015). Low load for disruptive mutations in autism genes and their biased transmission. *Proceedings of the National Academy of Sciences of the United States of America*.

[64] O’Roak B. J., Vives L., Girirajan S. (2012). Sporadic autism exomes reveal a highly interconnected protein network of de novo mutations. *Nature*.

[65] Kaischeuer V. M., Feenstra I., van Ravenswaaij-Arts C. M. A. (2008). Disruption of the TCF4 gene in a girl with mental retardation but without the classical Pitt-Hopkins syndrome. *American Journal of Medical Genetics, Part A*.

[66] Page S. C., Hamersky G. R., Gallo R. A. (2018). The schizophrenia-and autism-associated gene, transcription factor 4 regulates the columnar distribution of layer 2/3 prefrontal pyramidal neurons in an activity-dependent manner. *Molecular Psychiatry*.

[67] Rannals M. D., Hamersky G. R., Page S. C. (2016). Psychiatric Risk Gene Transcription Factor 4 Regulates Intrinsic Excitability of Prefrontal Neurons via Repression of SCN10a and KCNQ1. *Neuron*.

[68] Xia K., Guo H., Hu Z. (2014). Common genetic variants on 1p13.2 associate with risk of autism. *Molecular Psychiatry*.

The article "Integrative Functional Genomic Analysis in Multiplex Autism Families from Kazakhstan" was published in 2022. Journal: Dis Markers.

[69] De Rubeis S., He X., Goldberg A. P. (2014). Synaptic, transcriptional and chromatin genes disrupted in autism. *Nature*.

[70] Serajee F. J., Nabi R., Zhong H., Mahbubul Huq A. H. (2003). Association of INPP1, PIK3CG, and TSC2 gene variants with autistic disorder: implications for phosphatidylinositol signalling in autism. *Journal of Medical Genetics*.

[71] Deutsch S. I., Kreiser N. L., Urbano M. R., Burket J. A., Pickle J. C. (2017). Autism presenting in the context of a genetic variant of CFTR and early HSV exposure confounded by chronic pain, altered gut microbiota and paternal abandonment; limitations of current pharmacotherapy and barriers to personalized treatment recommendations. *Personalized Medicine in Psychiatry*.

[72] Chen C. H., Chen H. I., Chien W. H. (2017). High resolution analysis of rare copy number variants in patients with autism spectrum disorder from Taiwan. *Scientific Reports*.

[73] Cheng S. H., Gregory R. J., Marshall J. (1990). Defective intracellular transport and processing of CFTR is the molecular basis of most cystic fibrosis. *Cell*.

[74] Marcorelles P., Friocourt G., Uguen A., Ledé F., Férec C., Laquerrière A. (2014). Cystic fibrosis transmembrane conductance regulator protein (CFTR) expression in the developing human brain: comparative immunohistochemical study between patients with normal and mutated CFTR. *Journal of Histochemistry and Cytochemistry*.

[75] Caruso R., Warner N., Inohara N., Núñez G. (2014). NOD1 and NOD2: signaling, host defense, and inflammatory disease. *Immunity*.

[76] Al Nabhani Z., Dietrich G., Hugot J. P., Barreau F. (2017). Nod 2: the intestinal gate keeper. *PLoS Pathogens*.

[77] Jiang W., Wang X., Zeng B. (2013). Correction to recognition of gut microbiota by NOD2 is essential for the homeostasis of intestinal intraepithelial lymphocytes. *Journal of Experimental Medicine*.

[78] Jiang W., Wang X., Zeng B. (2013). Recognition of gut microbiota by NOD2 is essential for the homeostasis of intestinal intraepithelial lymphocytes. *Journal of Experimental Medicine*.

[79] Ogura Y., Bonen D. K., Inohara N. (2001). A frameshift mutation in NOD2 associated with susceptibility to Crohn’s disease. *Nature*.

[80] Robertson S. J., Geddes K., Maisonneuve C., Streutker C. J., Philpott D. J. (2016). Resilience of the intestinal microbiota following pathogenic bacterial infection is independent of innate immunity mediated by NOD1 or NOD2. *Microbes and Infection*.

[81] Petnicki-Ocwieja T., Hrncir T., Liu Y. J. (2009). Nod2 is required for the regulation of commensal microbiota in the intestine. *Proceedings of the National Academy of Sciences*.

The article "Integrative Functional Genomic Analysis in Multiplex Autism Families from Kazakhstan" was published in 2022. Journal: Dis Markers.

[82] Ramanan D., Tang M. S., Bowcutt R., Loke P., Cadwell K. (2014). Bacterial sensor Nod2 prevents inflammation of the small intestine by restricting the expansion of the commensal bacteroides vulgatus. *Immunity*.

[83] Valicenti-McDermott M. D., McVicar K., Cohen H. J., Wershil B. K., Shinnar S. (2008). Gastrointestinal symptoms in children with an autism spectrum disorder and language regression. *Pediatric Neurology*.

[84] Butwicka A., Olén O., Larsson H. (2019). Association of childhood-onset inflammatory bowel disease with risk of psychiatric disorders and suicide attempt. *JAMA Pediatrics*.

[85] el Turk J. (2022). Microbiome & autism spectrum disorders. *(IJRE) International Journal of Research and Ethics (ISSN 2665-7481)*.

[86] Kim J. Y., Choi M. J., Ha S. (2022). Association between autism spectrum disorder and inflammatory bowel disease: a systematic review and meta-analysis. *Autism Research*.

[87] Lim J. S., Lim M. Y., Choi Y., Ko G. (2017). Modeling environmental risk factors of autism in mice induces IBD-related gut microbial dysbiosis and hyperserotonemia. *Molecular Brain*.

[88] Lee M., Krishnamurthy J., Susi A. (2018). Association of autism spectrum disorders and inflammatory bowel disease. *Journal of Autism and Developmental Disorders*.

[89] Andersen A. B. T., Ehrenstein V., Erichsen R., Frøslev T., Sørensen H. T. (2013). Parental inflammatory bowel disease and risk of autism spectrum disorders in offspring: a nationwide cohort study in Denmark. *European Journal of Epidemiology*.

[90] ABT A., Ehrenstein V., Erichsen R., Frøslev T., Sørensen H. T. (2014). Autism spectrum disorders in children of parents with inflammatory bowel disease - a nationwide cohort study in Denmark. *Clinical and Experimental Gastroenterology*.

[91] Munton R. P., Vizi S., Mansuy I. M. (2004). The role of protein phosphatase-1 in the modulation of synaptic and structural plasticity. *FEBS Letters*.

[92] Hamdan F. F., Srour M., Capo-Chichi J. M. (2014). De novo mutations in moderate or severe intellectual disability. *PLoS Genetics*.

[93] Eneqvist T., Lundberg E., Nilsson L., Abagyan R., Sauer-Eriksson A. E. (2003). The transthyretin-related protein family. *European Journal of Biochemistry*.

[94] Goodman D. W. S. (1980). Plasma retinol-binding protein. *Annals of the New York Academy of Sciences*.

[95] Gião T., Saavedra J., Cotrina E. (2020). Undiscovered roles for transthyretin: from a transporter protein to a new therapeutic target for Alzheimer’s disease. *International Journal of Molecular Sciences*.

[96] Zhou L., Tang X., Li X., Bai Y., Buxbaum J. N., Chen G. (2019). Identification of transthyretin as a novel interacting partner for the *δ* subunit of GABA A receptors. *PLoS One*.

The article "Integrative Functional Genomic Analysis in Multiplex Autism Families from Kazakhstan" was published in 2022. Journal: Dis Markers.

[97] Coghlan S., Horder J., Inkster B., Mendez M. A., Murphy D. G., Nutt D. J. (2012). GABA system dysfunction in autism and related disorders: From synapse to symptoms. *Neuroscience and Biobehavioral Reviews*.

[98] Sesarini C. V. (2015). GABAergic neurotransmission alterations in autism spectrum disorders. *Neurotransmitter*.

[99] Rahnama M., Tehrani H. A., Mirzaie M. (2021). Identification of key genes and convergent pathways disrupted in autism spectrum disorder via comprehensive bioinformatic analysis. *Informatics in Medicine Unlocked*.

[100] Reilly J., Gallagher L., Leader G., Shen S. (2020). Coupling of autism genes to tissue-wide expression and dysfunction of synapse, calcium signalling and transcriptional regulation. *PLoS One*.

[101] Schwede M., Nagpal S., Gandal M. J. (2018). Strong correlation of downregulated genes related to synaptic transmission and mitochondria in post-mortem autism cerebral cortex. *Journal of Neurodevelopmental Disorders*.

[102] Mosca E., Bersanelli M., Gnocchi M. (2017). Network diffusion-based prioritization of autism risk genes identifies significantly connected gene modules. *Frontiers in Genetics*.

[103] Lorsung E., Karthikeyan R., Cao R. (2021). Biological timing and neurodevelopmental disorders: a role for circadian dysfunction in autism spectrum disorders. *Frontiers in Neuroscience*.

[104] Geoffray M. M., Nicolas A., Speranza M., Georgieff N. (2016). Are circadian rhythms new pathways to understand autism spectrum disorder?. *Journal of Physiology Paris*.

[105] Pinato L., Galina Spilla C. S., Markus R. P., da Silveira Cruz-Machado S. (2019). Dysregulation of circadian rhythms in autism spectrum disorders. *Current Pharmaceutical Design*.

[106] Nielsen J., Kulahin N., Walmod P. S., Berezin V. (2008). Extracellular Protein Interactions Mediated by the Neural Cell Adhesion Molecule, NCAM: Heterophilic Interactions Between NCAM and Cell Adhesion Molecules, Extracellular Matrix Proteins, and Viruses. *Neurochemical Research*.

[107] Petrovska J., Coynel D., Fastenrath M. (2017). The NCAM1 gene set is linked to depressive symptoms and their brain structural correlates in healthy individuals. *Journal of Psychiatric Research*.

[108] Vojdani A., Campbell A. W., Anyanwu E., Kashanian A., Bock K., Vojdani E. (2002). Antibodies to neuron-specific antigens in children with autism: Possible cross-reaction with encephalitogenic proteins from milk, Chlamydia pneumoniae and Streptococcus group A. *Journal of Neuroimmunology*.

[109] Lin Y. S., Wang C. C., Chen C. Y. (2021). Gwas meta-analysis reveals shared genes and biological pathways between major depressive disorder and insomnia. *Genes (Basel)*.

The article "Integrative Functional Genomic Analysis in Multiplex Autism Families from Kazakhstan" was published in 2022. Journal: Dis Markers.

[110] Smith I. A., Knezevic B. R., Ammann J. U. (2010). BTN1A1, the mammary gland butyrophilin, and BTN2A2 are both inhibitors of T cell activation. *The Journal of Immunology*.

[111] Ammann J. U., Cooke A., Trowsdale J. (2013). Butyrophilin Btn 2a2 Inhibits TCR activation and phosphatidylinositol 3-kinase/Akt pathway signaling and induces Foxp 3 expression in T lymphocytes. *The Journal of Immunology*.

[112] Rhodes D. A., Chen H. C., Price A. J. (2015). Activation of human *γδ* T cells by cytosolic interactions of BTN3A1 with soluble phosphoantigens and the cytoskeletal adaptor periplakin. *The Journal of Immunology*.

[113] Ashwood P., Wills S., van de Water J. (2006). The immune response in autism: a new frontier for autism research. *Journal of Leukocyte Biology*.

[114] Ohja K., Gozal E., Fahnestock M. (2018). Neuroimmunologic and neurotrophic interactions in autism spectrum disorders: relationship to neuroinflammation. *Neuromolecular Medicine*.

[115] Paysour M. J., Bolte A. C., Lukens J. R. (2019). Crosstalk between the microbiome and gestational immunity in autism-related disorders. *DNA and Cell Biology.*.

[116] Mazón-Cabrera R., Vandormael P., Somers V. (2019). Antigenic targets of patient and maternal autoantibodies in autism spectrum disorder. *Frontiers in Immunology*.

[117] Loayza M., Carter K., Pang Y., Bhatt A. J. (2020). Altered fetal microglia phenotypes are associated with abnormal neurogenesis following maternal immune activation. *Journal of Investigative Medicine*.

[118] Nadeem A., Ahmad S. F., Attia S. M., Al-Ayadhi L. Y., Al-Harbi N. O., Bakheet S. A. (2020). Dysregulation in IL-6 receptors is associated with upregulated IL-17A related signaling in CD4+ T cells of children with autism. *Progress in Neuro-Psychopharmacology and Biological Psychiatry*.

[119] Horiuchi F., Yoshino Y., Kumon H. (2021). Identification of aberrant innate and adaptive immunity based on changes in global gene expression in the blood of adults with autism spectrum disorder. *Journal of Neuroinflammation*.

[120] Braunschweig D., Van de Water J. (2012). Maternal autoantibodies in autism. *Archives of neurology*.

[121] Choi C. S. W., Souza I. A., Sanchez-Arias J. C., Zamponi G. W., Arbour L. T., Swayne L. A. (2019). Ankyrin B and Ankyrin B variants differentially modulate intracellular and surface Cav 2.1 levels. *Molecular Brain*.

[122] Iqbal Z., Vandeweyer G., van der Voet M. (2013). Homozygous and heterozygous disruptions of ANK3: at the crossroads of neurodevelopmental and psychiatric disorders. *Human Molecular Genetics*.

[123] Bi C., Wu J., Jiang T. (2012). Mutations ofANK3identified by exome sequencing are associated with Autism susceptibility. *Human Mutation*.

The article "Integrative Functional Genomic Analysis in Multiplex Autism Families from Kazakhstan" was published in 2022. Journal: Dis Markers.

[124] Balabanski L., Serbezov D., Atanasoska M. (2021). Rare genetic variants prioritize molecular pathways for semaphorin interactions in Alzheimer’s disease patients. *Biotechnology and Biotechnological Equipment*.

[125] Lindy A. S., Stosser M. B., Butler E. (2018). Diagnostic outcomes for genetic testing of 70 genes in 8565 patients with epilepsy and neurodevelopmental disorders. *Epilepsia*.

[126] O'Roak B. J., Deriziotis P., Lee C. (2011). Exome sequencing in sporadic autism spectrum disorders identifies severe de novo mutations. *Nature Genetics*.

[127] The Autism Spectrum Disorders Working Group of The Psychiatric Genomics Consortium (2017). Meta-analysis of GWAS of over 16,000 individuals with autism spectrum disorder highlights a novel locus at 10q24.32 and a significant overlap with schizophrenia. *Molecular Autism*.

[128] Wu J., Yu P., Jin X. (2018). Genomic landscapes of Chinese sporadic autism spectrum disorders revealed by whole-genome sequencing. *Journal of Genetics and Genomics*.

[129] López-Hernández T., Ridder M. C., Montolio M. (2011). Mutant GlialCAM causes megalencephalic leukoencephalopathy with subcortical cysts, benign familial macrocephaly, and macrocephaly with retardation and autism. *American Journal of Human Genetics*.

[130] López-Hernández T., Sirisi S., Capdevila-Nortes X. (2011). Molecular mechanisms of MLC1 and GLIALCAM mutations in megalencephalic leukoencephalopathy with subcortical cysts. *Human Molecular Genetics*.

[131] Guo H., Wang T., Wu H. (2018). Inherited and multiple de novo mutations in autism/developmental delay risk genes suggest a multifactorial model. *Molecular Autism*.

[132] Satterstrom F. K., Kosmicki J. A., Wang J. (2020). Large-scale exome sequencing study implicates both developmental and functional changes in the neurobiology of autism. *Cell*.

[133] Choi L., An J. Y. (2021). Genetic architecture of autism spectrum disorder: lessons from large-scale genomic studies. *Neuroscience and Biobehavioral Reviews*.

[134] Searles Quick V. B., Wang B., State M. W. (2021). Leveraging large genomic datasets to illuminate the pathobiology of autism spectrum disorders. *Neuropsychopharmacology*.

[135] Velinov M. (2019). Genomic copy number variations in the autism clinic—work in progress. *Frontiers in Cellular Neuroscience*.

[136] Chawner S. J., Doherty J. L., Anney R. J. (2021). A genetics-first approach to dissecting the heterogeneity of autism: phenotypic comparison of autism risk copy number variants. *American Journal of Psychiatry*.

[137] Shishido E., Aleksic B., Ozaki N. (2014). Copy-number variation in the pathogenesis of autism spectrum disorder. *Psychiatry and Clinical Neurosciences*.

The article "Integrative Functional Genomic Analysis in Multiplex Autism Families from Kazakhstan" was published in 2022. Journal: Dis Markers.

[138] Calle Sánchez X., Helenius D., Bybjerg-Grauholm J. (2022). Comparing copy number variations in a Danish case cohort of individuals with psychiatric disorders. *JAMA Psychiatry*.

[139] Wang Z., Diao C., Liu Y. (2019). Identification and functional analysis of GCK gene mutations in 12 Chinese families with hyperglycemia. *Journal of Diabetes Investigation*.

[140] Buchmayer S., Johansson S., Johansson A., Hultman C. M., Sparén P., Cnattingius S. (2009). Can association between preterm birth and autism be explained by maternal or neonatal morbidity?. *Pediatrics*.

[141] Allard L., Cochat P., Leclerc A. L. (2015). Renal function can be impaired in children with primary hyperoxaluria type 3. *Pediatric Nephrology*.

[142] Belostotsky R., Seboun E., Idelson G. H. (2010). Mutations in DHDPSL are responsible for primary hyperoxaluria type III. *American Journal of Human Genetics*.

[143] Fang X., He L., Xu G., Lin H., Xu M., Geng H. (2019). Nine novel HOGA1 gene mutations identified in primary hyperoxaluria type 3 and distinct clinical and biochemical characteristics in Chinese children. *Pediatric Nephrology*.

[144] Du Y., Roger V. B., Mena J., Kang M., Stoller M. L., Ho S. P. (2021). Structural and chemical heterogeneities of primary hyperoxaluria kidney stones from pediatric patients. *Journal of Pediatric Urology*.

[145] Riedel T. J., Knight J., Murray M. S., Milliner D. S., Holmes R. P., Lowther W. T. (2012). 4-Hydroxy-2-oxoglutarate aldolase inactivity in primary hyperoxaluria type 3 and glyoxylate reductase inhibition. *Biochimica et Biophysica Acta-Molecular Basis of Disease*.

[146] Konstantynowicz J., Porowski T., Zoch-Zwierz W. (2012). A potential pathogenic role of oxalate in autism. *European Journal of Paediatric Neurology*.

[147] Shattock P., Whiteley P. (2010). The role of oxalates in autism and chronic disorders. *Nutrition*.

[148] Pepin M., Schwarze U., Superti-Furga A., Byers P. H. (2000). Clinical and genetic features of Ehlers–Danlos syndrome type IV, the vascular type. *New England Journal of Medicine*.

[149] Schwarze U., Goldstein J. A., Byers P. H. (1997). Splicing defects in the COL3A1 gene: marked preference for 5’ (donor) splice-site mutations in patients with exon-skipping mutations and Ehlers-Danlos syndrome type IV. *American Journal of Human Genetics*.

[150] Casanova E. L., Baeza-Velasco C., Buchanan C. B., Casanova M. F. (2020). The relationship between autism and Ehlers-Danlos syndromes/hypermobility spectrum disorders. *Journal of Personalized Medicine*.

[151] Li F. Y., El‐Hattab A. W., Bawle E. V. (2010). Molecular spectrum of SLC22A5 (OCTN2) gene mutations detected in 143 subjects evaluated for systemic carnitine deficiency. *Human Mutation*.

The article "Integrative Functional Genomic Analysis in Multiplex Autism Families from Kazakhstan" was published in 2022. Journal: Dis Markers.

[152] Frigeni M., Balakrishnan B., Yin X. (2017). Functional and molecular studies in primary carnitine deficiency. *Human Mutation*.

[153] Guevara-Campos J., González-Guevara L., Guevara-González J., Cauli O. (2019). First case report of primary carnitine deficiency manifested as intellectual disability and autism spectrum disorder. *Brain Sciences*.

[154] Shi H., Wang J., Zhao Z. (2019). Analysis of inborn error metabolism in 277 children with autism spectrum disorders from Hainan. *Zhonghua Yi Xue Yi Chuan Xue Za Zhi= Zhonghua Yixue Yichuanxue Zazhi= Chinese Journal of Medical Genetics*.

[155] Beaudet A. L. (2017). Brain carnitine deficiency causes nonsyndromic autism with an extreme male bias: a hypothesis. *BioEssays*.

[156] Mayfield J. A., Davies M. W., Dimster-Denk D. (2012). Surrogate genetics and metabolic profiling for characterization of human disease alleles. *Genetics*.

[157] Zaidi S. H., Faiyaz‐Ul‐Haque M., Shuaib T. (2012). Clinical and molecular findings of 13 families from Saudi Arabia and a family from Sudan with homocystinuria. *Clinical Genetics*.

[158] Schiff M., Delorme R., Benoist J. F., Ogier de Baulny H. (2010). Faut-il faire un bilan métabolique dans l’autisme?. *Archives de Pediatrie*.

[159] Žigman T., Petković Ramadža D., Šimić G., Barić I. (2021). Inborn errors of metabolism associated with autism spectrum disorders: approaches to intervention. *Frontiers in Neuroscience*.

[160] Baralle D., Baralle M. (2005). Splicing in action: assessing disease causing sequence changes. *Journal of Medical Genetics*.

[161] Douglas J., Hanks S., Temple I. K. (2003). NSD1 mutations are the major cause of Sotos syndrome and occur in some cases of weaver syndrome but are rare in other overgrowth phenotypes. *American Journal of Human Genetics*.

[162] Türkmen S., Gillessen-Kaesbach G., Meinecke P. (2003). Mutations in NSD1 are responsible for Sotos syndrome, but are not a frequent finding in other overgrowth phenotypes. *European Journal of Human Genetics*.

[163] Kurotaki N., Imaizumi K., Harada N. (2002). Haploinsufficiency of NSD1 causes Sotos syndrome. *Nature Genetics*.

[164] Buxbaum J. D., Cai G., Nygren G. (2007). Mutation analysis of the NSD1 gene in patients with autism spectrum disorders and macrocephaly. *BMC Medical Genetics*.

[165] Rauch A., Thiel C. T., Schindler D. (2008). Mutations in the pericentrin (PCNT) gene cause primordial dwarfism. *Science*.

[166] Bober M. B., Niiler T., Duker A. L. (2012). Growth in individuals with Majewski osteodysplastic primordial dwarfism type II caused by pericentrin mutations. *American Journal of Medical Genetics, Part A*.

